This article has been retracted.

# Exploring the impact of climate technology, financial inclusion and renewable energy on ecological footprint: Evidence from top polluted economies

**DOI:** 10.1371/journal.pone.0302034

**Published:** 2024-04-18

**Authors:** Lu Wang, Fanyuan Ye, Jianlin Lin, Natasha Bibi

**Affiliations:** 1 School of Teacher Education, Nanjing University of Information Science and Technology, Nanjing, China; 2 Jiangsu Key Laboratory for Optoelectronic Detection of Atmosphere and Ocean, Nanjing University of Information Science & Technology, Nanjing, China; 3 Business School, The University of Sydney, Sydney, NSW, Australia; 4 College of Electrical Engineering, Shanghai University of Electric Power, Shanghai, China; 5 Business School, Virtual University, Lahore, Pakistan; University of Pitesti, Romania; Institute of Doctoral and Post-doctoral Studies, University Lucian Blaga of Sibiu, ROMANIA

## Abstract

Most South Asian countries’ economies have grown dramatically during the past few decades. However, in light of their environmental sustainability goals, the quality of such growth performances by South Asian nations is called into doubt by the concurrent degradation in environmental quality. Consequently, reducing the environmental challenges these nations encounter is prioritized on the agendas of the relevant authorities. This study aimed to analyze the effect of the top 11 most polluted countries’ levels of financial inclusion, technological innovation, consumption of renewable energy, and adoption of climate technology on environmental deterioration from 2000 to 2022. Therefore, this research aims to use cutting-edge panel data econometric techniques to investigate the factors contributing to high carbon footprints in the world’s most polluted nations. The results support an inverted U-shaped relationship between economic growth and carbon footprints, crediting the environmental Kuznets curve concept. In addition, it has been shown that TECH, REC, and CT can reduce carbon footprints in both the short and long term, while GDP and financial inclusion only affect carbon footprints in the long term. The results further endorsed the pollution haven hypothesis by showing that GDP positively affects carbon footprint. As a result, leading polluting economies need to strengthen their financial sectors, create green technology, migrate to renewable energy, and limit financial inclusion to improve environmental quality.

## Section 1: Introduction

A worldwide trend toward using cleaner technology to slow the rate of global warming has resulted from the formulation of sustainable development goals (SDGs) set by the United Nations. Nations have been directed by the international agreement to keep GW below 2 degrees Celsius, with 1.5 degrees C being preferable [1]. It is communal practice to use emissions of (CO_2_) and (GHG) as proxies for the effect of business and consumption on ecological quality. But it’s necessary to have a sweeping indicator considering all the major environmental deterioration factors. In this context, EFP is a reliable indicator for measuring the ecological effects of human actions. Agricultural, pasture, and forest lands, as well as built-up and carbon demand on land, are all factors that EFP considers, making it a helpful indicator [2].

The Environmental Kuznets Curve (EKC) method stands out in environmental discourse because it provides the theoretical underpinnings for tackling the drivers of environmental degradation. The EKC hypothesis was first future by Fareed et al. [3], who argued that financial development has negative effects on the atmosphere. According to the EKC hypothesis’s theoretical explanation, a rise in per capita income first hastens environmental degradation before slowing pollution emissions. Due to their massive economic and industrial activity, high-growth economies must pay the opportunity costs of environmental deterioration [4]. The EKC hypothesis states that beyond a certain point, GDP reduces environmental strain while further expansion increases it. A nation’s ability to embrace pollution abatement techniques, such as green innovation projects, importing state-of-the-art industrial systems, and modernizing antiquated systems, increases when its GDP rises above a specific threshold. All of these actions will lead to cleaner air in the long run, as predicted by the U-shaped relationship. The EKC hypothesis has been empirically linked to a wide range of variables in numerous researches [5].

The size of a nation’s ecological footprint is said to be heavily influenced by its trade and GDP levels. This is because they reveal insights on the nation’s production and consumption habits. The pace of industrialization and the expansion of global trade are common yardsticks by which producers measure their output. The relationship between trade policies and environmental impact often varies between developing and wealthy nations. Since most developing republics are tranquil in the early periods of their financial development, they are often forced to adopt technologies that are not environmentally friendly while mass producing goods. Furthermore, these nations’ reliance on fossil fuels to encounter energy weights puts stress scheduled current incomes and pushes the biocapacity bound to its absolute maximum. However, industrialized countries have moved previous this stage then is additional likely toward implement trade policies that encourage technological advancement and increase reliance arranged REN resources. The EFP of every country is directly impacted by its foreign and domestic trade activity, including exports and imports. When this is considered, it is easy to see how trade contributes to environmental damage. When comparing CO_2_ emissions in Italy between 1995 and 2009, Hassan et al. [6] find that the majority are tied to imports rather than exports.

Furthermore, when the banking industry is thriving, it is easy for people and enterprises to secure the financing they need. The demand for machinery, technological equipment, and cars in the industrial and transportation sectors rises alongside financial inclusion, worsening environmental conditions as a result of increased energy [7]. Several current educations model the social, economic and environmental nexus through agriculture, energy use, financial development, EG and forests [8]. This is done to specify that financial and agriculture development may assistance in explaining differences in environmental footmark and CO_2_ releases planes. Scale, composition, and method effects may influence environmental footmark and CO_2_ emissions as an effect of innovations in agriculture, financial inclusion, and FDI [9]. Small shifts in these factors, especially in light of the scale effect, can have large effects on productivity, greenhouse gas and energy use emissions. On the further indicator, the composition effect illustrates how an economy shifts its focus to producing products after their relationship gain, which stimulates the expansion of financial and agricultural sectors and may vary emissions depending on whether or not the nation resumes manufacturing goods and services that are energy-exhaustive. The use of energy-intensive production techniques could improve ecological security due to the method effect, which describes the spread of technology through the movement of agricultural and monetary development from country to country. Similarly, if an industry’s financial system is robust, it may invest more in cutting-edge technology, which, in turn, increases energy consumption. Finance innovation may also lead to greener corporate practices and a smaller carbon footprint [10].

For the purposes of this study, EFP was chosen as the environmental performance indicator. Biologically productive areas that can either perpetually create incomes or dispose of anthropogenetic wilds are referred to as having an "ecological footprint" [11]. The following arguments support using environmental footmark as the indicator of ecological presentation in this investigation. At its core, sustainable development’s ecological evaluation can be summed up by the concept of the environmental footprint, which measures humankind’s environmental effect in relation to the resilience of the Earth’s bio system. It’s a crucial indicator for gauging progress toward the SDGs [12]. Second, the ability to absorb wastes is crucial to ecological sustainability. Minerals, trees, soil, and water are all put to productive use in today’s economy. Pollutants as a metric fail to account for these factors; as a result, EFP appears to be a more comprehensive indicator [13]. Humanity’s " EFP " illustrates the pressure humans place on ecosystems and establishes a link between consumption and the biosphere’s capacity for renewal [14]. It’s a more all-encompassing measure of ecological decline and economic viability than individual metrics like, GHGs, carbon emissions, and other contaminants [15].

This being the case context, the existing examine seeks to study the effect of RNE use, energy transition, financial development and environmental innovation on EFP in the context of top ten manufacturing economies experiencing macro regressors such as economic growth and urbanization. Environmental difficulties in manufacturing products or providing services are included in the biological footmark EFP [16]. Included are forest land, pasture land, agriculture land, ocean area, carbon footprint and developed land. The EFP is the sole metric that explains the gap between human consumption and regenerative capacity [17].

For the purposes of this study, ecological footprint was chosen as the environmental performance indicator. Biologically productive areas that can either perpetually create dispose or resources of anthropogenetic wastes are referred to as having a "biological footmark" [18]. The following arguments support using EFP as the indicator of ecological act in this investigation. At its core, sustainable development’s ecological evaluation can be summed up by the idea of leaving a "footprint" on the environment, which measures humankind’s environmental effect in relation to the resilience of the Earth’s bio system. It’s a crucial indicator for gauging progress toward the SDGs [12]. Second, the ability to absorb wastes is crucial to ecological sustainability. Minerals, trees, soil, and water are all put to productive use in today’s economy. Pollutants as a metric fail to account for these factors; as a result, environmental footmark appears for a better comprehensive indicator [19]. Humanity’s " EFP " illustrates the pressure humans place on ecosystems and establishes a link between consumption and the biosphere’s capacity for renewal [20]. Compared to isolated metrics like carbon emissions, GHGs, and other pollutants [21], it is a more thorough indication of environmental degradation and economic viability. The detrimental effects of climate change and environmental degradation on the global ecological environment have attracted a lot of attention in recent years [22]. Fossil fuels are the key factors that produce GHG emissions and cause environmental deterioration, according to a number of recent research [23]. According to our research on the energy consumption patterns of the world’s top 10 manufacturing nations, fossil fuels continue to play a significant role. In 2019, the United States produced roughly 4.12 trillion kWh of energy, of which RNE accounted for only 17.5% (720 kW h), whereas natural gas accounted for 38.4% (1582 kW h), and oil accounted for 62.7% (2580 kW h). As a result, greenhouse gas emissions due to energy use have increased by 2.7%, or 5130 MMT.

This study goals to examine the environmental, energy, and other key variables in 11 emerging nations from 1990 to 2021. Nevertheless, the present study enhances the existing body of literature in the following manners. 1) This study has included the impact of TECH on EFP. The primary reason for this is the recognition that the contemporary world is transitioning towards a novel model of manufacturing and consumption, which will ultimately necessitate a more intelligent utilization of existing resources. Hence, the notion of sustainable development is intricately connected to the capacity of states to meet the resource needs of present societies without detrimentally impacting future generations. The number of patent applications in emerging economies has significantly increased from 0.11 million to 1.74 million between 1980 and 2016. Li et al. [24] contend that by appropriately acknowledging and valuing technical advancements, sustainable growth can be attained through the effective utilization of natural resources. Therefore, global economies can effectively address the limited availability of valuable natural resources and fulfill the demands of a growing population by leveraging technology advancements, while minimizing any additional harm to the environment. The shift from conventional technologies to eco-friendly technologies, such as reprocessing, recycling, implementing innovative processes, and utilizing alternative products, will result in economic growth and ultimately alleviate environmental degradation [25]. Hence, sustainable development is attained by means of TECH, industrial conversion, and the advancement of RNE sources to diminish reliance on fossil fuels, thereby facilitating economic and social progress. This is particularly applicable when evaluating a win-win scenario that promotes both economic growth and environmental conservation.

Similarly, the current study likewise employs environment-related technology as a pivotal determinant of EFP. The existing literature suggests that although there have been numerous studies on the environmental impacts of technologies in various national contexts, there is a scarcity of research examining the contribution of environmental-related technologies to the EFP. Therefore, further investigation is warranted in this area. In addition, existing literature frequently employs carbon emissions as a metric for assessing environmental deterioration, but the EFP is seen as a more encompassing measure [26]. The empirical results do not definitively establish the long-term positive effect of environmental-related technologies on carbon footprint reduction. Nevertheless, the positive impact of green technologies on the EFP is not observed in the stated economies. The empirical findings also suggest that a comprehensive approach that encompasses the interconnected variables of environment, technology, and economic growth is required to effectively address the concerns and establish a sustainable environment. These findings suggest that certain policy implications should be considered in order to promote the advancement and implementation of environmentally-friendly technology, with the aim of achieving sustainable development goals.

Financial inclusion (FIN) has garnered significant interest in the environmental literature because to its potential to alleviate excessive environmental burdens at the home level. This study is the first to analyze the influence of foreign investment (FI) on environmental footprint (EFP) in the chosen economies. This is important since these economies are experiencing rapid economic expansion, which poses a risk to global environmental sustainability. The findings of our research have significant ramifications for policymakers in economies that are concerned about achieving ecologically sustainable growth. These policymakers aim to promote economic expansion while simultaneously mitigating ecological degradation, in line with the region’s objective of meeting the Sustainable Development Goals by 2030. Therefore, this limitation is resolved by using EFP, a complete measure for environmental sustainability [27]. Hence, doing thorough research will not only broaden the existing knowledge base but also offer profound insights for the formulation of policies aimed at attaining sustainable development objectives. Thus, the utilization of the EFP distinguishes this study from previous investigations. Furthermore, we plan to enhance the extensive utilization of RNE sources in certain economies is highly valued. The study’s main contribution lies in its suggested scheme, which has the potential to restore the ecological system and address the long-standing issue of environmental pollution, all while ensuring economic growth remains undisturbed. The suggested method has the potential to significantly reduce both economic and environmental costs by utilizing nonrenewable resources at the industrial and home levels, without causing employment loss. Hence, it would constitute a pioneering addition to the current body of literature [5].

In light of this context, it is crucial to investigate of the correlation between economic growth and EFP. Hence, this study examines the correlation between EG and ecological impact in the context of the nation’s swift advancement. This study addresses a significant research gap in the existing literature by being the first to investigate the primary factors that determine the EFP of specific economies. Moreover, certain economies have become signatories of the Kyoto agreement inside the framework of the United Nations. This work utilizes tests for CSD, as well as second-generation unit root tests, cointegration tests, and estimation, in order to avoid inaccurate estimations that may result from ignoring CSD among countries. Furthermore, the key empirical approaches applied include CS-ARDL, AMG, CCEMG, and FMOLS. These methods offer indisputable factual proof to assist in the formulation of eco-friendly policies.

Following is a plan for the remainder of the research: Literature reviews are discussed in Section 2. Data description, theoretical context, and empirical technique are presented in Section 3. The empirical findings are described in Section 4. Conclusions and suggestions for further action are provided in Section 5.

## Section 2: Literature review

Similarly, this section is divided into three different subsections such as 1) Nexus of Climate technology and Environmental Degradation; 2) Nexus of Financial Inclusion with Environmental Degradation; 3) Nexus of Renewable Energy and Environmental Degradation.

### 2.1. Nexus of Financial Inclusion with Environmental Degradation

The literature extensively investigates the potential factors that influence environmental quality, particularly the EFP and other relevant indicators, as well as the significance of environmental-related technology. Divergences in the empirical data characterize the existing body of research, which can be largely categorized into three categories. The first set of data is based on associations between eco-friendly technology and well-known indicators of environmental health, like carbon and emissions of greenhouse gases (GHG). In his study covering the years 1999–2015, Liu et al. [28] looks at 20 OECD nations and how their carbon emissions, environmental policy stance, and green technology adoption rates all interacted. Environmental laws and development both have a long-term influence on lowering CO_2_ emissions, according to the empirical data. Consistent with this idea, Kebede et al. [29] found that, for OECD economies, eco-patents and logos reduced carbon emissions from 1990 to 2015. Two recent studies by OECD researchers examine how energy R&D affects GHG emissions: Wang et al. [30] and Burchi et al. [31]. The results show that technological and energy innovations mitigate the detrimental consequences of energy intensity on the environment. From 1990 to 2017, the G7 countries’ CO₂ emissions were studied by Cai and Wei [32]. Environmental innovation and diversification of exports were the subjects of the research. In accordance with the data, export diversification raises CO₂ emissions while environmental innovation lowers them. When innovation levels rise, however, export diversification’s detrimental impact is minimized. The impact of technological progress on environmental sustainability has been found to be either negligible or even negative, according to other studies. Luo et al. [33] argue that OECD countries have achieved a point of extreme technological advancement, which is apparently causing a rebound effect on carbon emissions. A similar finding and criticism of innovation as the principal source of carbon emissions in 24 OECD nations are reported by Naor et al. [34]. Banna et al. [35] analyze the effect of scale, combined, and technological factors on OECD countries’ carbon emissions. They conclude that technological progress does not significantly help in cutting carbon emissions through making energy efficiency better. Down their 2020 study, Danish and Ulucak zero down on the developing nations of the BRIC to examine the link between environmentally friendly inventions, renewable and non-renewable energy sources, and green economic growth across the years. Environmental technology and renewable energy have been crucial in promoting sustainable economic growth, according to the empirical estimates produced from panel data covering the years 1992–2016. The effect of eco-friendly technologies on reducing emissions of greenhouse gases and carbon dioxide (CO_2_) in the E7 nations is evaluated in the research by Chuc et al. [36]. These results provide credence to the idea that renewable energy sources and technology focused on the environment can help achieve long-term sustainability goals. When it comes to the effect of RNE and technological advancements on carbon levels in Next-11 nations, there has been very little study. Green technologies and renewable energies significantly reduce CO_2_ emissions over lengthy periods of time, according to authors using dataset covering 1980–2018. However, improvements brought about by environmentally friendly technology do not materialize right away. Du et al. [37] examine, with a focus on the effects of technological developments, the connection between CO_2_ emissions in China and investments in public-private collaboration in the energy sector. The situation within China is the particular focus of the investigation. While technical progress helps to lessen environmental externalities, the empirical results show that public-private partnership investment significantly degrades environmental quality. On the other hand, Ojo [38] look at 70 countries’ responses to climate change via the lens of innovation from 1976 to 2014. The ability of a country to innovate and create climate change technology is correlated with its levels of greenhouse gas (GHG) emissions, according to empirical data. Climate technology innovation is not necessarily a byproduct of government initiatives in areas like energy, telecoms, transportation, and environmental projects.

Also, a more all-encompassing measure, EFP, has replaced traditional environmental quality indicators in recent years. The Environmental Kuznets Curve (EKC) theory is examined in 15 European nations by [39]. There is a notable difference between the empirical results obtained using DOLS and FMOLS, two econometric methods. Although the latter method suggests that this is true for some countries, the former method’s estimation results show that there is a U-shaped association between affluence and EFP in other nations. In their 2020 study, Altintas and Kassouri test the validity of the EKC hypothesis using data from 14 European nations spanning 1990–2014. The two writers offer a new take on EFP as an important indicator of environmental health. Both the EKC theory and the beneficial effects of renewable energy on the environment are backed up by the actual results. The elements that contribute to the environmental imprint in developing nations have been the subject of numerous studies. The factors that influence the environmental impact of BRICS countries are investigated by Menkeh et al. [40]. It was found that the three parts—urbanization, renewable energy, and rent from natural resources—had a good impact on the environment. Data from real-world experiments back up the EKC theory. Tsimisaraka [41] look at eleven newly industrialized nations to see if the EKC theory is correct. A curvilinear association, with an inverted U-shape, among GDP and EFP is supported by the panel data that spans from 1977 to 2013. Among eight oil-exporting nations in the Middle East and North Africa region, Ahmad et al. [42] found an inverse U-shaped association between actual wealth and EFP. Interestingly, in seven nations that do not produce oil for export, the relationship between actual wealth and environmental impact takes the form of a U-shaped curve. Energy use, urbanization, and EG all have an effect on the EFP of the Next-11 nations, which Koomson et al. [43] analyze. While urbanization does lead to environmental decline in most countries, it can be mitigated by examining how income and urbanization interact. This connection can significantly reduce environmental degradation. In Pakistan, Baskaya et al. [44] look at how bio-capacity, EG, and environmental effect are related. In terms of EFP, the data show that these factors significantly contribute to environmental degradation. Tsimisaraka et al. [41] use a larger dataset to test the EKC hypothesis in high-, medium-, and low-income economic groups. There is a positive association between income and the EFP in the beginning, but this relationship weakens as economies develop.

Thirdly, using two bodies of literature, the group delves into the environmental impact of green technology to determine its EFP. However, a dearth of in-depth studies on the use of eco-friendly technology to control environmental impact has been identified, particularly in OECD nations. By using a panel dataset that includes BRICS countries from 1993 to 2017, Tsimisaraka et al. [42] are able to measure the short-term and long-term effects of environmental technology and institutional quality on the EFP. According to the numbers, the BRICS countries’ governments are strengthening their structures to deal with environmental issues. On the other hand, it’s smart to push for green tech investments, since these can lessen the environmental toll. A panel dataset that includes 22 developing nations and covers the years 1984–2016 is used by Le et al. [45]. They intend to look into the relationships between ecological impact, rent from natural resources, technological advancement, and economic activity. According to the statistics, technical innovation is one of the best ways to lessen negative impacts on the environment. Jia et al. [46] examined the impact of technological advancements on the environmental impact and carbon emissions of key developing nations. Technological advancements may lessen CO_2_ emissions, but they do nothing to aid in environmental footprint management.

### 2.2. Nexus of Financial Inclusion with Environmental Degradation

Within the framework of environmental protection and financial inclusion (FIN), recent studies have sought to identify the elements that lead to sustainable growth. The findings, however, differ among the research nations in relation to their income and developmental stage. A number of contexts are examined in this study, including MINT countries Eton et al. [47], developing countries [48], countries that are part of the Kyoto annex [49], Sri Lanka [50], China [51], and South East Asian economies. Reducing pollution levels is one way a healthy financial system helps bring in FDI. In addition, innovative ideas and technology to lower emissions of greenhouse gases are encouraged by improving finance systems. On the flip side, researchers looked into the connection between carbon dioxide emissions and FIN using panel data from 31 Asian economies from 2014 to 2017. An index representing FIN was constructed using principal component analysis (PCA). The research shows that expanding access to financial services has negative effects on the natural world. One factor that has been identified as adding to the environmental impacts of the top 20 carbon-emitting economies is financial inclusion, which is also called financial development. The EKC hypothesis was shown to be unsupported by the panel data in the bidirectional study. Further, it was discovered that energy usage and financial inclusion both contribute to smaller environmental footprints. Additionally, energy consumption adds to the rise of GDP, but FIN has a good effect on environmental preservation, according to Alvarado et al. [52]. This study develops its working hypothesis by expanding upon these ambiguous arguments.

The relationship between financial inclusion and economic advancement has been the subject of scholarly debate among several researchers. Recent years have seen an expansion in the amount of written work by academics concerned with the external effects that the financial sector may have on the world’s natural resource base. Additionally, the link between environmental protection and FIN has been the subject of more and more debate. Determining if FIN develops, degrades, or has no effect on environmental quality is the most controversial subject. The use of different proxies, estimate methodologies, panels (countries), and time periods measured in the research causes the large variances in these linkages. From 2004 to 2014, Adedoyin et al. [53] looked at how many factors such inclusive finance, urbanization, FDI, energy consumption, and industrialization affected global warming in Asian countries. Rising energy demand and easier access to financial services are major threats to environmental sustainability, according to the experts. In addition, the relationship between FIN and environmental deterioration in the OIC states was investigated by [53]. They argue that reducing emissions of greenhouse gases is one of the many benefits of expanding access to financial services. For China, Wang and Zhang [54] found similar results, and Burger and Calitz [55] found similar results for Tunisia and Pakistan, respectively. On the other hand, a lot of academics think that financial inclusion could help with reducing carbon emissions. One effective strategy for reducing carbon emissions is financial inclusion, which facilitates the adoption of cutting-edge low-carbon solutions by businesses. There is an inverse relationship between economic growth and carbon dioxide emissions, according to research by Cao et al. [56]. Financial inclusion and the alleviation of energy poverty were the foci of Zhao et al. [57] research. They found that eliminating energy poverty is within reach because to Ghana’s fast increase of FIN. Research has shown that FIN can decrease carbon emissions by reducing energy poverty. FIN directly affects the decrease of CO_2_ emissions, according to the empirical evidence provided by Khan et al. [58]. Beyond the obvious direct relationship, there may be a more indirect relationship between inclusive finance and environmental performance. The inverse U-shaped connection among financial inclusion and carbon emissions was examined by Díaz et al. [59] using a panel of 103 nations. Validation of the EKC from 1990 to 2017 was carried out by Khowaja et al. [60] across various South Asian nations. It appears that economic growth reduces CO_2_ emissions in the long run, even while it increases emissions in the short term. In their 2019 study, Ren et al. [61] verified that the EKC hypothesis holds water in APEC member nations. This assertion is backed by other studies done in 2018 by Ren et al. [61]. The link between FIN and environmental performance is unclear, though. A further point is that the significance of financial inclusion in helping to attain the SDGs has been acknowledged. There may be positive and negative effects of financial inclusion on sustainability performance.

### 2.3. Nexus of Renewable Energy and Environmental Degradation

The relationship between energy use, environmental deterioration, and economic expansion has been the subject of numerous articles. There are mainly three types of these studies. A major focus of the research is the relationship between energy utilization and GDP. The correlation between energy use and GDP growth has also been the subject of a great deal of published work. A plethora of research pertaining to static and dynamic econometric analysis, with a focus on different nations, has emerged since the 1978 publication by these studies [62–66]. However, the study’s empirical findings show that the direction of causation differs among nations. Using Hsiao’s Granger causality test, Shang et al. [67] looked at the data from 1960–2001 to see how Turkey’s GDP and energy use were related. The factors in question do not appear to be causally related. On the other hand, a study investigating the direct relationship between energy usage and economic expansion in Algeria’s economy from 1971 to 2010 was carried out by Rehman et al. [68]. A two-way causal relationship between the variables is shown by the VECM analysis. Using panel regression analysis, Doğan et al. [69] found that fossil energy usage—more especially coal energy—had a positive and substantial effect on the economic growth of the BRICS economies between 1995 and 2014.

The second set of researchers looked at the correlation between rising prices and emissions of carbon dioxide, a measure of environmental deterioration. The Environmental Kuznets Curve (EKC) is associated with it, and it implies that the relationship between GDP growth and CO_2_ is inverted U-shaped. Corrosion and pollution, according to the EKC theory, are more prevalent during the beginning phases of EG, but then they start to decline once income levels reach a certain point. When income levels are raised, the environment benefits from economic growth. According to Ali et al. [70], pollutants in the environment indices are inversely related to economic growth. Grossman and Krueger were the ones that first proposed the EKC idea. Countless other investigations using the EKC architecture followed. This includes works by authors such as Mendoza-Del Villar et al. [71] and Jabeen and Khan [72]. Results from empirical investigations testing the EKC hypothesis disagree, even when looking at the same geographical areas.

The third grouping brings together the first two to look at how renewable and non-renewable energy usage relate to economic growth, environmental degradation (including EFP), and energy consumption overall. In recent years, a great deal of research has focused on how changes in trade and finance, EG, and energy utilization affect EFP. From 1971 to 2014, the environmental impacts of developing nations were studied by Hu et al. [73]. They looked at how consumption of energy, urbanization, and economic expansion affected these impacts. Based on the results, it seems that urbanization is good for the environment. Next-11 nations see less environmental degradation and a smaller EFP as a consequence of urbanization and economic expansion working together to offset this effect. The purpose of Tang et al. [74] research is to analyze how six factors—urbanization, emissions of carbon dioxide, agricultural land usage, fishery ground exploitation, woodland usage, and grazing land usage—converge to form a person’s EFP. The research incorporates information from 92 countries and spans 54 years, beginning in 1961 and ending in 2014. According to the results, there are four convergence groups for the built-up footprint and ten for the EFP. There are five convergence clubs that deal with carbon footprints, seven that deal with footprints on agriculture, and two that deal with footprints on fishing grounds. They discover two convergence clubs for pastures footprint and find total convergence for forest land footprint. Two convergence clubs for EFP were found in the post-merging investigation, but six convergence clubs for cropland footprint were identified.

What effects do renewable and fossil fuel energy sources have on the environment? Samargandi et al. [75] looked into it. Using 74 economies’ data sets spanning 1990–2015, the researchers used panel causality and FMOLS approaches. There is a negative and statistically significant coefficient for green energy consumption, in contrast to the expanding influence of fossil fuel use on environmental degradation, according to the empirical evidence. According to the writers, pollution levels are going up since the financial sector is growing. Additionally, they verified that the EKC theory was correct for the nations in question. Between 1996 and 2012, Tongurai and Vithessonthi [76] studied 25 developing economies to determine the correlation between RNE usage, GDP, and international commerce. Increasing the share of RNE consumption leads to a considerably bigger drop in carbon emissions, according to the study that used DOLS and fractional maximum override (FMOLS) methods. But long-term CO_2_ emissions rise as green energy consumption scales up. The environmental impact is positively affected by trade. In addition, the EKC concept has been validated by their empirical data. Salari et al. [77] investigated the relationship between Qatar’s environmental impact, financial sector development, yield, and trade openness using the Markov Switching Equilibrium Correction Model (MS-ECM). Over the period from 1970 to 2015, he revealed the constant equilibrium between all of these factors. In addition, he found that EFP and yield are cause and effect relationships, and that power consumption and total foreign trade are one-sided causalities that lead to EFP. His research established a direct causal relationship between EFP and economic development. The EKC hypothesis was tested for 116 nations by Tariq et al. [78] using data collected between 2004 and 2008. By examining the EFP’s import and production components, the study proved that the EKC theory is valid. In addition, panel regression analysis demonstrated that higher energy uses per capita led to lower production footprint and higher imported footprint. Researchers Isik et al. [79] tested the EKC hypothesis across fifteen MENA nations. For countries that exported oil between 1975 and 2017, the researchers found that the theory was correct. A U-shaped correlation, however, was observed for non-oil exporting countries. On top of that, according to the results of the panel FMOLS and DOLS investigations, energy consumption reduced the EFP, whereas urbanization increased it. From 1971 to 2016, Zainal et al. [80] studied the effects of hydroelectric energy usage on the environment in Malaysia. Using parameters like EFP, water footprint, carbon footprint, and carbon dioxide emissions, they have developed four separate models. Using hydroelectric power reduced environmental deterioration, according to the ARDL border test, whereas increased urbanization increased it. Furthermore, they confirmed that the EKC theory was credible with respect to Malaysia. In their 2019 study, Elshimy and El-Asar looked at six Arabic countries to see how income, livestock, and energy sources affected carbon footprint. From 1980 to 2014, the researchers analyzed data using Panel FMOLS and DOLS Models. There is evidence in Arab nations for the EKC concept, according to empirical studies. An additional 0.14% reduction in carbon footprint is achieved with a 1% increase in RNE sources. Still, the increased use of non-renewable energy sources causes a 0.35% increase in the carbon footprint, while the expansion of livestock raises the carbon footprint by 0.42%. To determine how renewable energy sources affect environmental effect, Purnamawati [81] used a panel research. In their analysis, they used the FMOLS and DOLS techniques. The data set used in the study covers the years 1992–2016, with a particular emphasis on the BRICS nations. All countries’ environmental Kuznets curve (EKC) hypotheses were confirmed by the economic calculations. It has also been found that natural resource preservation, renewable energy use, and urbanization all help to lessen the environmental impact. Zhao et al. [82] examined 22 nations in Central and South America and found that pollution has increased over time in correlation with trade and economic levels. Conversely, things that contribute to improved environmental quality include renewable energy sources, more tourism, and foreign direct investments. The purpose of the study by Aurangzaib and Farooq [83] was to examine the relationship between South Africa’s per capita energy use, income, and environmental impact. From 1973 to 2014, the researchers analyzed the association between income and environmental deterioration using the bound test and Toda-Yamamoto causality analysis. Their research shows that the accumulation of wealth contributes to environmental damage over time. Energy consumption is the main factor affecting the EFP, and over a long period of time, there is a negative association between the two. From 1977 to 2013, researchers Gwani and Sek [84] looked at eleven nascent industrialized nations to determine the relationship between energy usage and environmental impact. For South Africa, the Philippines, Mexico, and Singapore, the Augmented Mean Group (AMG) analysis backs up the EKC theory. Nevertheless, the link between Turkey, China, India, South Korea, and Thailand is formed like a U. In addition, panel causality analysis has proven that energy use is the main cause of the environmental impact.

### 2.4. Research gap

After looking over the mentioned literature, it’s clear that previous studies didn’t do a good job of investigating the link between the EFP and resource use. Few studies have shown conflicting findings. Possible explanations for the contradictory findings include different methods of extracting resources, different administrative processes, and unique national traits. In order to create an effective environmental strategy to combat climate change, technological progress is essential. However, carbon dioxide (CO_2_) emissions have been the primary focus of the extant literature on the impact of technological breakthroughs on environmental degradation. A thorough comprehension of this major problem cannot be achieved by discussing climate change with a singular focus on CO_2_ emissions. Using the EKC as a framework, this study investigates the short- and long-term relationships between natural resource depletion, technological progress, economic growth, and changes in the EFP. The natural resources of the globe are largely in the hands of emerging nations, and their rate of development is outpacing that of industrialized nations [85]. Therefore, it’s vital to look at how the aforementioned components are related in developing economies too.

## Section 3: Data and modeling approach

### 3.1. Data

The empirical investigate draws on information on 11 developing nations from 1990 to 2022 (China, Brazil, India, Nigeria, Mexico, Bangladesh, Russia, South Africa, Pakistan, Turkey, and Vietnam). This study analyzes how financial inclusion and Technological innovation have affected Brazil’s environmental impact. The model also considers variables like GDP, FIN, and TECH. EFP is the dependent variable, whereas GDP, FIN, TECH, CT, and REC are the exogenous variables. The origin, direction, and units of measurement for the variables under study are all listed in Table 1 and Fig 1. In addition, the natural logs of all the investigation’s variables are taken to guarantee their normality.

**Fig 1:** Scatter plot of the selected variables.

**Table 1:** Variables of the study.

Description of the variable	Symbol	Measurement unit	Source
Ecological Footprint	EFP	Measured in terms of constant per capita	GFN
Technological innovations	TECH	Number of environmental patents per year	IRENA
Climate Technology	CT	Environment-related technologies	OECD
Financial Inclusion	FIN	The FIN index is a metric that quantifies the accessibility, comprehensiveness, and effectiveness of financial services.	IMF database
Renewable energy consumption	REC	Total, % of primary energy supply	WDI
Economic growth	EG	GDP per capita (2015 US$)	WDI

Authors’ Elaboration

#### 3.1.1. Ethical approval and consent to participate

The authors declare that they have no known competing financial interests or personal relationships that seem to affect the work reported in this article. We declare that we have no human participants, human data or human tissues.

### 3.2. Econometric models

In this study, four models have been used. These models are given in Eqs (1–4).

**Model-I:**

$${\text{EFP}}_{i,t}=f\left(EG_{i,t},TECH_{i,t}CT_{i,t},FIN_{i,t},REC_{i,t}\right)$$ 1

**Model-II:**

$${\text{EFP}}_{i,t}=f\left(EG_{i,t},{\text{TECH}}_{i,t}{\text{CT}}_{i,t},{\text{FIN}}_{i,t},REC_{i,t},{\left(TECH*FIN\right)}_{i,t}\right)$$ 2

**Model-III:**

$${\text{EFP}}_{i,t}=f\left(EG_{i,t},TECH_{i,t}CT_{i,t},FIN_{i,t},REC_{i,t}{\left(CT*FIN\right)}_{i,t}\right)$$ 3

**Model-IV:**

$${\text{EFP}}_{,i,t}=f\left(EG_{i,t},TECH_{i,t}CT_{i,t},FIN_{i,t},REC_{i,t},{\left(REC*FIN\right)}_{i,t}\right)$$ 4

### 3.3. Econometric modelling approach

In order to determine how dependent, the variables are, the CSD test is run first. A unit- The root-testing procedure is employed to if panel data are stationary. Next, we utilize the SH test to establish if the model is heterogeneous or homogeneous. The following stage is to conduct a panel analysis of cointegration to establish whether or not the variables are interrelated across time. In addition, the CS-ARDL test is used to evaluate both the immediate and longstanding effects of the variable star in the econometric approach. The results’ dependability on the, sample selection, model specification and other parameters are examined in a robustness test.

#### 3.3.1. Cross-sectional dependence test

When (N) is big, it is conventional in piece data models to suppose that disturbances are cross-sectionally independent. Panel regression, however, has been proven in a large number of studies to exhibit cross-sectional dependency (CSD). Relative reliance can have a significant impact on the efficiency and test statistics of an estimate if it is not considered. Scaled LM, bias-corrected scaled LM, and CSD are used to evaluate CSD. The following are representations of (H_0_) and (H_1_) applicable to the CSD test (See Eq 5):

$${\text{H}}_{0}:\rho_{ij}=Cov\left(\mu_{it},\mu_{it}\right)=0,noCSD$$ 5

$${\text{H}}_{1}:\rho_{ij}=Cov\left(\mu_{it},\mu_{it}\right)\neq 0,yesCSD$$

The slightly revised CSD test [86] is given by Eqs (6) and (7). It is suggested that this variant be used with unbalanced panels.


$$CSD_{P}=\sqrt{\frac{2T}{N(N-1)}}\left(\sum_{i=1}^{N-1}\sum_{j=i+1}^{N}\rho_{ij}\right)∼N(0,1)\text{i},\text{j}$$ 6

$$R=\sqrt{\frac{2T}{N(N-1)}}\left(\sum_{i=1}^{N-1}\sum_{j=i+1}^{N}{\hat{\rho }}_{ij}\right)\left[(T-k)\frac{{\hat{\rho }}_{ij}^{2}-(T-k){\hat{\rho }}_{ij}^{2}}{\text{Var}(T-k){\hat{\rho }}_{ij}^{2}}\right]$$ 7

Since the model was assessed with fixed-effects cross-sectional for developing nations, the biased corrected LM statistic was also computed. Using Eq. (8), we can utilize the Lagrange multiplier exam statistic to identify correlations and dependances in CSD [87].


$$CSD_{BP}=\sum_{i=1j=i+1}^{N-1}\sum_{ij}^{N}{\hat{\rho }}_{ij}^{2}\to \chi^{2}\frac{N_{\left(N-1\right)}}{2}$$ 8

It has long been known that the CSD of Pagan and Breusch (1980), where the default test statistic in LM is set to *CSD*_*BP*_, is inadequate for testing in large populations. [88] suggests an improved version of the Lagrange multiplier statistic (CSD LM), as indicated in Eq (9), as a possible solution to this issue. The scaled LM test statistic provided by [29] is shown to benefit from a straightforward asymptotic bias correction in Eq (10).


$$CSD_{LM}=\sqrt{\frac{1}{N(N-1)}}\sum_{i=1j=i+1}^{N-1}\sum_{ij}\left(T_{ij}{\hat{\rho }}_{ij}^{2}-1\right)\to N(0,1)$$ 9

$$CSD_{BC}=\sqrt{\frac{1}{N(N-1)}}\sum_{i=1j=i+1}^{N-1}\sum_{ij}^{N}\left(T_{ij}{\hat{\rho }}_{ij}^{2}-1\right)-\frac{N}{2(T-1)}\to N(0,1)$$ 10

In Eqs (7), (8), (9), and (10), the term ${\hat{\rho }}_{ij}^{2}$ applies an OLS regression to explore paired cross-sectional correlations.

#### 3.3.2. Unit-root test

Incorporating the Panel Unit Root Test, Third Generation, Was Developed By [27], which builds on the extensive improvements proposed by [28], who included providing evidence of dependency within the context of testing for unit roots in panels, we find that the former provides better empirical relevance and utility. The [89] statistic is provided by Eq (11), and a modified Sargan-Bhargava (MSB) test is performed across numerous series using a data pooling strategy.


$$\text{MSB}=\frac{T^{-2}\sum_{t=1}^{T}{\hat{e}}_{t-1}^{2}}{{\hat{\sigma }}^{2}}$$ 11

Where ${\hat{e}}_{t}$ is a consistent estimator, and ${\hat{\sigma }}^{2}$ represents the estimated residuals. Three pooling statistics, *Z* (the standardization of the individual statistics), *P*, (the product of the p values), and *P*_*m*_ (the product of the p values), provide three distinct test statistics when multiple structural disruptions for respectively sequence and mutual data apparatuses are included. The fundamental specification is given in Eq (12), and the reliability of the infinite-sample tests has been verified using [35].


$$\log\left(\frac{p_{i}}{1-p_{i}}\right)=\sum_{j=0}^{1}\left(\zeta_{0j}+\zeta_{1j}q\left(p_{i}\right)+\zeta_{2j}q{\left(p_{i}\right)}^{-\frac{1}{2}}+\zeta_{3j}q{\left(p_{i}\right)}^{-\frac{1}{3}}+\zeta_{4j}q{\left(p_{i}\right)}^{-\frac{1}{4}}\right){\left(\frac{1}{T_{i}}\right)}^{j}+u_{i}$$ 12

#### 3.3.3. SH test

The slope homogeneity (SLH) among the cross-sections is evaluated once the CSD has been calculated. Disparities in the economic and demographic bases of the BRI countries make the issue of heterogeneity more pressing. Panel estimator reliability could be affected by varying the slope parameters. Because of this, the SLH method was utilized $\tilde{\Delta }$ test [90]: we use the test of [89], which is founded on the modified [91] statistic $\tilde{S}$, which is suitable in the instance of *N*,*T*→∞ (See Eqs (13 and 14):

$$\tilde{\Delta }={\left(N\right)}^{\frac{1}{2}}{\left(2K\right)}^{-\frac{1}{2}}\left(\frac{1}{N}S-k\right),$$ 13

$${\tilde{\Delta }}_{adj}={\left(N\right)}^{\frac{1}{2}}{\left(\frac{◂\cdot ▸\;2k(T-k-1)}{T+1}\right)}^{-\frac{1}{2}}\left(\frac{1}{N}S-k\right)$$ 14

#### 3.3.4. Panel cointegration test

The panel cointegration test [91]was performed after the SH test and the unit-root test were completed. However, Wu et al. [91] (all first-generation techniques for cointegration) have produced skewed results because of variation in the size properties. As a result, during the research, a set of panels cointegration tests. The essential goal of these examines is to verify the existence of a causal association among the variable quantity for each of the developing nations. The purpose of the analysis is to examine unit root tests with residuals, differentiate it with the use of shared variables, and account for structural breaks. The goal of this research is to verify the locations of each cross-section’s breaks using an estimator of break sites. The core model can be expressed using the notation of Eqs (15) and (16).

$$y_{it}=\beta_{i}+\delta_{i}t+\gamma_{i}D_{it}+x_{it}^{\prime }\alpha_{i}+{\left(D_{it}x_{it}\right)}^{\prime }\rho_{i}+Z_{it}$$ 15

$$x_{it}=x_{it-1}+\xi_{it}$$ 16

where and T represent the time series and cross-section, correspondingly; and illustrates the structurally-aware time imitation. Which stands for the intercept and slope before the structural breaks, respectively, are compared with which stands for the intercept and slope after the structural breaks, in order to examine situations in the market that are volatile. The two forms of cointegration tests used in this study are the coefficient test and the t-test version, both of which can be seen as extensions of the LM unit root tests (Eqs (17) and (18)). Both of the examinations are outlined here. Even when applied to limited datasets, the findings of these two experiments hold water.


$${\text{LM}}_{\phi }=-{\left(2\int_{0}^{1}U_{i}{\left(s\right)}^{2}\text{d}s\right)}^{-1}$$ 17

$${\text{LM}}_{\tau }=-{\left(4\int_{0}^{1}U_{i}{\left(s\right)}^{2}\text{d}s\right)}^{-1/2}$$ 18

Uddin et al. [92] and kassi et al. [93] used common correlated effects estimator (CCE), which assumes that A unifying factor is most adequate for modeling cross-sectional dependencies, to conduct similar research into the cointegrating relationship between variables. These parameters can be estimated using cross-sectional averages of the model variables. Correct test regression Eq (20) is obtained by adding these means to the right-hand side of Eq (19):

$$y_{it}=\alpha_{i}+\beta_{i}^{\prime }{\text{x}}_{it}+\epsilon_{it}$$ 19

where α is a slope coefficient vector unique to that member, and β is a fixed effect unique to that member.


$$y_{it}=\alpha_{i}+\beta_{i}^{\prime }{\text{x}}_{it}+\lambda_{i}\bar{{\text{z}}_{t}}+v_{it}$$ 20

The stochastic regressors and the dependent variable both have cross-sectional averages that are kept in the vector ${\bar{z}}_{t}={\left({\bar{y}}_{t},{\bar{x}}_{t}^{\prime }\right)}^{\prime }\;\text{is}\;\text{a}(m+1)\times 1.$ The model is estimated using the Pooled CCE estimator, and residual stationarity is verified afterwards. The method works within the framework of spurious regression and can handle, non-stationary, heterogeneity, panel data, weak and strong CSD, and admirable limits.

#### 3.3.5. CS-ARDL test

The present study used the robust estimate technique of cross-sectional increased autoregressive distributive lag (CS-ARDL) [94] to calculate both short ‐ and long -term outcomes. The study used the CS-ARDL method, which has important advantages over regular econometric models due to the study’s strong assumptions about unobserved heterogeneity, cross-country dependency and variable endogeneity. In addition, this method excels in T > N scenarios, as the one examined here. The main benefit of the CS-ARDL technique is that it achieves consistent statistics regardless of the integration order of the underlying variables by modeling the long-run implications in the equation and integrating the effects of unobserved components. Therefore, khan et al. [58] implemented the CCE method of [95] in the context of board ARDL models, where the lag of the reliant on variables was treated as a weakly exogenic variable inside the fault alteration framework. By incorporating cross-section averages of the dependent and independent variables affected by these unobserved mutual shocks and the related insulated values of these variables, the CS-ARDL method corrects for the unobserved consequences of common shocks, expanding the conventional ARDL strategy. To estimation the research classical in Eq (1), the panel CS-ARDL follows the economy as shown by the Eq (21):

$$y_{i,t}=\alpha_{i}+\sum_{j=1}^{p}\lambda_{ij}y_{i,t-j}+\sum_{j=0}^{q}\delta_{ij}^{\prime }x_{i,t-j}+\sum_{j=0}^{k}\varphi_{ij}^{\prime }{\bar{Z}}_{i,t-j}+\varepsilon_{it}$$ 21

K represents the lag duration and is the residual, which includes the unnoticed joint components that cause dependence between cross-sectional units; $\bar{Z}={\left({\bar{y}}_{i},{\bar{x}}_{i}\right)}^{\prime }$ represents a comparison of the means of ${\bar{y}}_{i}$) the dependent variable and (${\bar{x}}_{i}$) the independent variable across a sample size n.

The results from CS-ARDL were put to the test by using two alternative estimate strategies: Peseran’s mutual correlated effect mean group (CCEMG) [96] and Eberhardt and Bond’s augmented mean group (AMG) [97]. In order to properly supplement the CS-ARDL estimator results, the CCEMG and AMG assessment tools generate efficient and trustworthy statistics in CSD heterogeneous panels.

#### 3.3.6. Causality test

As a last step in the empirical research, we use the Hurlin and Dumitrescu causality test to investigate the connection among the independent and dependent variables. When dealing with cross-sectional and heterogeneity dependence, this method outperforms the granger causality test. It is also applicable in cases when N is smaller than or equal to T, in addition in imbalanced panels. The econometric form of the DH test is as follows:

$$Y_{it}=\varphi_{i}+\sum_{k=1}^{K}\tau_{i}^{\left(k\right)}Y_{i,t-k}+\sum_{k=1}^{K}\delta_{i}^{\left(k\right)}X_{i,t-k}+\varepsilon_{i,t}$$ 22

In Eq 22, K and *φ*_*i*_ represent the intercept and lag length, respectively; $\delta_{i}^{\left(k\right)}$ couriers the slope coefficient; $\delta_{i}=\delta_{i}^{\left(1\right)},\delta_{i}^{\left(2\right)}\ldots .,\delta_{i}^{\left(k\right)}$ is used to characterize the lag parameter; and $\delta_{i}^{\left(k\right)}$ and $\tau_{i}^{\left(k\right)}$ tell the story of differences across cross-section units. The alternative hypothesis describes the presence of at least one cross-section with a causal link, while the null hypothesis denies the incidence of such a connotation.

## Section 4: Results and discussion

### 4.1. Preliminary test results

We carefully examine descriptive examination to better understand the characteristics of the variables. The variables’ means, minimums, and maximums, as well as the differences between them, are all summarized in Table 2, together with other descriptive statistics about the underlying series. The normal and peak distribution pattern of the variables are shown in Table 2 with the use of the Jarque-Bera (JB) and kurtosis tests, correspondingly TR, GTI, REN, EFP, and GDP average out to be 1.623, 2.067, 1.149, 2.167, 3.929, and 10.363, respectively. When compared to other metrics, GDP and TR have greater means. Standard deviation, however, shows that REN is the most extreme., environmental taxation, green technology innovation, renewable energy use, EFP, economic development and trade openness, all exhibit a helpful trend, as seen in Table 2.

**Table 2:** Descriptive statistics.

Parameters	EFP	EG	TECH	CT	FIN	REC
**Mean**	4.056	12.924	5.892	3.053	7.062	3.951
**Min.**	2.162	10.675	1.875	1.829	3.342	2.93
**Max.**	7.589	16.864	7.692	4.247	7.666	1.354
**Std. Dev.**	2.523	2.679	2.831	4.944	1.063	5.073
**Skew.**	0.565	–1.466	–0.304	1.214	1.235	1.672
**Kurt.**	4.235	5.23	3.976	1.818	3.096	0.842

Source: Authors’ Calculation.

### 4.2. CSD test results

Given the interconnected nature global population economies for this reason of social and economic cooperation, the experiential technique of the present inquiry commences with testing of cross-sectional requirement. Because of this, it’s possible for the underlying impacts in one economy to ripple across to others., Pesaran LD, and Pesaran CD The Breusch-Pagan LM tests were selected to determine if there was any cross-sectional dependence. Table 3 shows that the given empirical findings support the presence of CD, with the majority of variables being significant at the 1% level and the remainder being significant at the 5% level.

**Table 3:** CSD test results.

	CSD_BP_		CSD_LM_		CSD_BC_		CSD_P_	
Variables	Stat.	*P-*Value	Stat.	*P-*Value	Stat.	*P-*Value	Stat.	*P-*Value
EFP	512.572*	0.00	54.669*	0.00	51.632*	0.00	22.289*	0.00
TECH	1244.490*	0.00	90.679*	0.00	85.626*	0.00	56.869*	0.00
CT	680.356*	0.00	92.361*	0.00	91.820*	0.00	45.394*	0.00
FIN	424.158*	0.00	63.876*	0.00	53.034*	0.00	18.637*	0.00
REC	1393.955*	0.00	127.090*	0.00	111.931*	0.00	38.554*	0.00
EG	2267.665*	0.00	239.743*	0.00	186.026*	0.00	66.627*	0.00

Note:

* directs the significance level at 1%.

### 4.3. Unit-root test results

The SH and CSD in Table 4 Panel-B and Panel-A are serious issues in panel data estimates that provide misleading and inconsistent outcomes. When relying on macroeconomic indicators, CSD is to be expected. The interdependence of national economies is often to blame for CSD. Consequently, the economies of neighboring countries are likewise affected by actions in one country. Because of the panel data’s variability, as indicated by the results of the SH test, suggests that the coefficients in the model are heterogeneous and that the slope differs among economies, as shown in Panel-B. It also demonstrates that the social and economic structure of one country cannot have a reciprocal effect on the other [98].

**Table 4:** Outcomes of unit root test.

Parameters	*Z*		*P*_*m*_		*p*	
	I(0)	I(1)	I(0)	I(1)	I(0)	I(1)
EFP	0.202	–4.515*	0.691	5.207*	21.108	75.107*
TECH	0.286	–3.945*	0.652	9.774*	22.370	61.423*
CT	0.400	–4.604*	0.287	6.847*	20.854	72.536*
FIN	0.186	–3.990*	0.658	8.649*	22.054	69.678*
REC	0.335	–3.101*	0.312	5.575*	18.464	63.876*
EG	0.644	–3.613*	0.174	5.664*	18.680	70.664*

Note:

*shows 1% significance level.

### 4.4. SH test results

To detect CSD and SH in our panel, we use the CSD test [99] and the SLH test [99]. Panel-A of Table 5 shows that CSD is present under our model’s assumptions; we also see that the values p for all the parameters are less than 0.001, indicating that we should discard the null hypothesis that there is no CSD. It suggests that the panel countries may be similarly affected by an economic shock in any variable in any one of the panel countries. The presence of heterogeneity in the panel data is shown in Panel-B of Table 5. Both models with EFP as a dependent variable have heterogeneous slopes, as shown by the SLH test, refuting the null hypothesis that the slope is homogenous. Due to the presence of CSD and heterogeneity, it is important to apply the second-generation unit root and second-generation cointegration [97] approaches to the panel data.

**Table 5:** SH test results.

SH test		Model I	Model II	Model III	Model IV
**Delta**	Stat.	29.654*	25.432*	26.221*	26.015*
	*P-*value	0.0000	0.0000	0.0000	0.0000
**Adjusted Delta**	Stat.	32.221*	21.325*	23.006*	22.923*
	*P-*value	0.0000	0.0000	0.0000	0.0000

Note:

*shows 1% significance level.

### 4.5. Panel cointegration test results

As part of this study, the cointegration test developed by Qin et al. [100] was implemented to look at the structural cracks that allow for CSD to happen. The results shown in Table 6 show that EFP, EG, TECH, CT, and FIN are cointegrated. This study employs a cointegration test developed by Banerjee and Carrion-i-Silvestre to look for evidence of a long-run relationship between two variables, and it also uses residual-based tests for panel cointegration with structural breaks and level shifts in the cointegrating association developed by Pata et al. [101] to see if there is, in fact, such a relationship near the location where the linear trend line has been broken. Table 6 shows that the null hypothesis is banned for all three trend factors (non-deterministic, constant, and trend), demonstrating that panels are cointegrated. There is a one percent statistically important change among the entire sample and individual countries.

**Table 6:** Cointegration test results.

Westerlund and Edgerton, (2008)				
Statistics	LM_T_	P-Value	LM*_ϕ_*	P-Value
No-Shift	–4.3510*	0.0000	–4.2119*	0.0000
Mean-Shift	–4.8725*	0.0000	–3.6924*	0.0000
Regime-Shift	–3.8276*	0.0000	–3.7362*	0.0000
**Banerjee and Carrion-i-Silvestre (2017)**				
Economies	**No deterministic specification**		**With constant**	**With trend**
Full Sample	–4.544*		–3.810*	–6.184*
Bangladesh	–5.023*		–5.134*	–5.809*
Brazil	–4.786*		–6.852*	–3.955*
China	–4.423*		–5.005*	–8.381*
India	–6.282*		–5.812*	–6.648*
Mexico	–5.968*		–5.633*	–7.672*
Nigeria	–4.243*		–5.419*	–7.058*
Pakistan	–4.660*		–4.675*	–8.236*
Russia	–4.578*		–6.032*	–8.424*
South Africa	–5.704*		–6.327*	–7.688*
Turkey	–5.367*		–6.717*	–8.068*
Vietnam	–5.371*		–4.969*	–7.234*

Note:

*shows 1% significance level.

At 5% and 10% constant, and at -2.92 and -2.82 with trend, the CV values are -2.32 and -2.18, respectively.

### 4.6. CS-ARDL test results

We used CS-ARDL as our primary econometric strategy, analyzing both the long-term and short- effects of the three standard econometric models (see Table 7). The long-term correlation between EG, TECH, CT, REC, EFP and FIN has been confirmed by the empirical coefficients. In all three models, we find that EFP is inversely related to our energy transition, primary variable, this indicates that environmental deterioration will be reduced in the world’s top 11 manufacturing countries as they make the switch from fossil fuels to renewable, eco-friendlier alternatives. In order to help achieve the low-carbon or zero-carbon targets established by a number of environmental agreements [15] policymakers, economic experts, and organizations have altered the environmental legislation process in recent years. Green economy is boosted and environmental problems are solved as a result of the shift to renewable energy sources [18]. We urge policymakers to place greater emphasis on the parts of the energy transition that contribute to the decoupling process on the basis of this evidence. Decoupling carbon emissions from industrial operations will be possible if energy transformation is prioritized in leading industrial economies. Similar statistical results were presented by [102, 103].

**Table 7:** CS-ARDL test results.

Model		Short-run		Long-run			
	Variables	Coeff.	t-stats.	*P* value	Coeff.	t-stats.	*P* value
**Model I**	TECH	–0.0923*	–3.4372	0.0004	–0.0915*	–3.9135	0.0005
	CT	–0.0874**	–2.6332	0.0011	–0.1720**	–2.7070	0.0013
	FIN	0.0723**	2.7342	0.0010	0.1955*	3.4955	0.0006
	REC	–0.2811*	–3.8156	0.0003	–0.1923	–4.9046	0.0000
	EG	0.1422*	4.3271	0.0000	0.2920*	4.9509	0.0000
	ECM (-1)	–0.6342*	–4.6342	0.0000	0.000	0.000	–
**Model II**	TECH	–0.1386**	–2.3658	0.0011	–0.5534	–3.9714	0.0000
	CT	–0.1833***	–1.6129	0.0136	–0.1735**	–2.5443	0.0014
	FIN	0.2822**	2.6659	0.0010	0.1561**	2.5560	0.0013
	REC	–0.3393*	–3.5172	0.0000	–0.3130*	–3.8367	0.0000
	EG	0.153*	4.6743	0.0000	0.2923*	6.4248	0.0000
	TECH * FIN	–0.1081*	–4.6587	0.0000	–0.2559*	–6.6580	0.0000
	ECM (-1)	0.7882*	3.9864	0.0000	0	0	–
**Model III**	TECH	–0.4298**	–2.1053	0.0013	–0.8235**	–2.3227	0.0014
	CT	–0.0856***	–1.8754	0.0020	–0.0474***	–1.8527	0.0231
	FIN	–0.0672**	–2.6252	0.0011	0.3341**	3.1365	0.0010
	REC	0.2143*	3.2421	0.0000	–0.2573*	–3.5984	0.0000
	EG	0.1281*	3.3232	0.0002	–0.4276*	3.9209	0.0000
	CT*FIN	–0.1433*	–4.5989	0.0000	–0.2336*	–6.1857	0.0000
	ECM (-1)	–0.2452**	–2.3213	0.0014	–	–	–
**Model IV**	TECH	0.0529**	2.0912	0.0015	–0.7047**	–2.1175	0.0016
	CT	–0.0982*	–3.654	0.0000	–0.0336*	–3.9527	0.0000
	FIN	0.1896**	3.9801	0.0000	0.2238**	3.8337	0.0000
	REC	–0.2534*	–4.2212	0.0000	–0.2800*	–4.0460	0.0000
	EG	–0.1618*	–4.6423	0.000	0.2670	5.0256	0.000
	REC* FIN	–0.1812*	–4.9743	0.0000	–0.3255*	–6.3128	0.0000
	ECM (-1)	–0.3832**	–3.5854	0.0000	–	–	–

Note:

*p<0.05

**p<0.10

***p<0.01

Approximations from a long-term panel model fit show that EG has a constructive effect on environmental footmark across the study period (1990–2022). This encouraging result indicates that the EFP is increasing in tandem with per capita GDP growth in these eleven developing countries. More specifically, in the short run, a 1% increase in real income per capita growth diminishes ecological prominence by 0.2781%, and in the long run, by 0.1422%. Some studies [104] find similar positive effects of GDP per capita growth on environmental footmark. Since these rising economies are among the fastest-growing in the world, and their economic development has increased dramatically over the past four decades, it is plausible to assume that their EG has had a positive effect on their increasing EFP. Increases in real per capita income have spurred increased investment across the board. Because of this, these developing nations now have the biggest EFPs and are major energy consumers. The estimated results also suggest that the link among environmental scarcity and income growth is weakened in these economies due to poor income per capita growth and weak ecological standards. An increase in economic output and an increase in energy intensity lead to a decrease in energy efficiency, as shown by the positive correlation. These results demonstrate the failure of ecological methods and policies to reduce the EFP that developing nations generate as their per capita wealth rises. However, the positive connection of GDP with EFP is validated by recent studies across the different regions, such as the case study of Pakistan economy [105], the case study of Emerging Market [106] and the study of China [107].

In addition, across all of the regression models, we find a negative relationship between EFP and the consumption of RE. It has been found that in developing nations, the coefficient for REC is significantly negative for EFP (-0.2811%). Increased acceptance of RNE sources in emerging nations is indicative of efforts to limit ecological degradation. REC and environmental issues are discussed from a variety of angles, and several authors share their unique insights. It is widely held that the environmental impression of REC is lower [108]. The estimated results are consistent with the previous studies by [109, 110], all of whom confirmed that the REC is helpful in reducing EFP. However, up to this point, developing nations have increased their use of RNE sources, which are clean and help reduce EFPs. From 2005 to 2016, emerging economies implemented roughly 197 separate renewable energy-based projects, contributing about 0.084 Giga tons of CO_2_ emissions to the overall decline of GHG emissions [111]. Deploying renewable energy helps reduce environmental impact by replacing fossil fuels and other nonrenewable energy sources with renewable ones. As a result, reducing the ecological influence of developing nations requires the Increasing reliance on renewable sources of energy. However, the negative association with ecological footprint or green energy can be supported by recent studies such as [112].

All empirical models show a negative and statistically important association among technical innovation and EFP. The fact that environmental degradation has been steadily decreasing over the past few years is evidence that this correlation holds true. The environmental pressure that results from the fact that industrial economies’ excessive push for economic progress is a leading contributor to environmental degradation is expected to further encourage those thrifts to embrace TECH and seek out alternative energy sources. As the pro-development agenda in the world’s top ten manufacturing countries coincides with environmental goals, it is clear that technological innovation will be bolstered by progress in the energy sector. Multiple studies corroborate our results, including those by Anshika et al. [111]. However, the current outcomes are in line with the case studies of the United States, the stud of BEM economies.

There is much discussion on the environmental effects of FIN. Similar to EFP, the correlation between FIN is positive and statistically significant. The long-term improvement in environmental quality due to a 1% influence on FIN is 0.35 percentage points for EFP and 0.32 percentage points for EFP. This suggests that FIN in BRI countries has a negative impact on ecological health. Kartiko et al. [113] state that a country’s emissions are proportional to its EG and FIN. Given these findings, it’s clear that FIN contributes to a higher overall pollution rate and more EFP pressure in BRI economies. Similar findings were found by Mendonça et al. [114], who hypothesized that easier access to financial services would boost industrial and commercial activities, which in turn would increase pollution. The growing growth of industrialization and transportation activity, along with the long-term project funding for 11 emerging economies, may increase demands on NRS. Increased resource exploitation, waste production, and environmental deterioration are all made possible by the alterations to economic growth prompted by financial deals. It encourages research and development and the financial industry at the expense of the environment. There has been a lot of focus on finding solutions to climate change and global warming and improving ecological sustainability. Similarly, these outcomes can be verified via some recent studies such as study of China by Juergensen. et al. [112], and the study of Ghana.

The long-term projections in Table 7 are reliable with the short-term results. For instance, an inverse relationship exists between EFP and energy transition, ecological innovation, and RNE because of the rising popularity of environmentally friendly technology, the accessibility of alternative energy sources, and the necessity of combining environmental and energy improvements to attain environmental sustainability. However, the concentration on financial reforms to pursue economic agendas worsens environmental quality in the top 11 manufacturing economies, and EFP is promoted as a transition towards becoming an advanced industrial economy.

### 4.7. Robustness analysis results

Table 8 shows the outcomes of the robustness estimation of the CS-ARDL estimations using the CCEMG and AMG estimators. Results from the CS-ARDL long-run estimates are similar to those from the CCEMG and AMG models, and the signs of the estimates are the same across a range of significance levels. Results for TECH and CT from the CCEMG and AMG confirm those from the CS-ARDL, which helps to improve ecological quality. Similarly, results from FIN, EG and REC reaffirm the worrying influence these metrics have on EFP in selected countries.

**Table 8:** Robustness test results.

Models	Parameters	CCEMG		AMG	
		Coeff.	t-stat.	Coeff.	t-stat.
**Model I**	TECH	–0.3694*	6.3348	–0.3243*	–3.5539
	CT	–0.1594**	3.0273	–0.1569**	–2.2581
	FIN	0.2935*	4.4808	0.2883*	3.4867
	REC	–0.1818*	4.3374	–0.1083*	–3.8031
	EG	0.1836*	4.6938	0.1730*	2.9550
**Model II**	TECH	–0.213**	3.4984	–0.1756**	–2.4532
	CT	–0.2602**	3.4689	–0.0342*	–3.9763
	FIN	0.0963*	7.9873	0.0546*	4.5434
	REC	–0.2611*	4.6308	–0.2341*	–2.9198
	EG	0.3768*	4.4508	0.1887*	3.7812
	TECH * FI	–1.4871**	3.0181	–1.8522**	–2.1452
**Model III**	TECH	–0.1815*	5.1198	–0.2151*	–3.8232
	CT	–0.2808	4.9074	–0.1653*	4.9823
	FIN	0.1330	7.3128	0.0872*	4.6241
	REC	–1.3666	5.7937	–0.9726*	–3.5421
	EG	0.3271*	4.1433	0.1911*	3.6342
	CT * FIN	–0.4822*	5.3464	–0.5430*	–4.9862
**Model IV**	TECH	–0.2733	5.6734	–0.3212*	–3.6723
	CT	–0.1771	5.3116	–0.1562*	5.8921
	FIN	0.0490	6.7638	0.1072*	4.8540
	REC	–1.0728	5.8876	–0.5541*	–3.5621
	GDP	0.4816	5.5131	0.5321*	3.1410
	REC * FIN	–0.6798***	11.784	–0.1875*	–6.8645

Note:

*p<0.05

**p<0.10

***p<0.01

### 4.8. Causality test results

The experimental results of Dumitrescu and Hurlin’s causality study are presented in Table 9; they show, at the 5% and 10% levels of significance, that there is a bidirectional causal link between EG and EFP in the top 11 polluted countries. REC, CT, TECH, EG, and FIN all have major effects on EFP, as shown by a causal analysis of these factors. Inferences can be drawn about the importance of EFP, the REC, and other variables in the study’s model for influencing the results of ecological policies in the world’s top 11 polluted economies. [115–118] all offer similar statistical findings. Further study results are expressed in Fig 2.

**Fig 2:** Variables relationship.

**Table 9:** Causality test results.

H_0_	W-stat.	t-stats.	*P*-value	Remarks
EG ⇎ EFP	5.360*	4.347	0.0010	EG ⟺ EFP
EFP ⇎ EG	4.055*	4.049	0.0000	
TECH ⇎ EFP	2.831**	2.348	0.0510	TECH ⟺ EFP
EFP ⇎ TECH	4.466*	3.739	0.0000	
CT ⇎ EFP	8.178***	2.832	0.0601	CT ⟺ EFP
EFP ⇎ CT	4.156***	2.502	0.0650	
FIN ⇎ EFP	4.420*	4.129	0.0400	FIN ⟺ EFP
EFP ⇎ FIN	3.532*	3.551	0.0020	
REC ⇎ EFP	6.069*	6.735	0.0000	REC ⟺ EFP
EFP ⇎ REC	2.839**	3.300	0.0480	

Note:

*p<0.05

**p<0.10

***p<0.01. ⟺ shows bidirectional causality

## Section 5: Conclusion and policy recommendations

The current study proposes significant policy implications for polluted economies to address the environmental burden. Initially, findings indicate that technological innovation is a significant factor of environmental degradation in economies with high levels of pollution. In line with these results, policymakers and central authorities should generate additional employment possibilities through research and development initiatives. As development progresses, the governments of these nations should form consortia to exchange perspectives and ideas in order to growth the use of clean energy sources. They should also promote energy efficiency and technological advancements. This include the implementation of stringent environmental regulations, advocating for ecologically conscious and adaptable policies, and employing appropriate technologies to mitigate environmental repercussions. The improvement of emission abatement TECH and the implementation of stringent ecological rules are crucial for reducing pollution levels. Policymakers in very polluted economies should be required to implement stringent measures if enterprises and consumers fail to comply with legislative endeavors aimed at reducing their EFP. These nations should also start adopting innovative policies and technologies that promote ecologically sustainable methods of invention. By doing so, individuals will have the ability to generate a sustainable level of employment that leads to an improvement in living conditions. The outcomes of this enhancement in living conditions will not only alleviate social disparities but also reduce income inequality. The government of Polluted economies should recognize the necessity to address the misalignment between technical advancements, cleaner technologies, and environmental regulations in order to effectively reduce the ecological imprint. If these conditions continue, the increasing pollution caused by industrialization would pose a threat to world sustainability. Therefore, it is crucial to establish a collaborative platform (consortia) to enhance and strengthen planning and coordination, research and development collaboration, and collective efforts towards cleaner innovation. This platform will also facilitate country-level exchanges, enable the sharing of eco-friendly technology, and initiate engineering, scientific, and enterprise alert ventures. The prevailing mindset of prioritizing pollution before treatment should be replaced with a mutually beneficial approach, where both economic growth and environmental quality are prioritized. This necessitates a shift away from relying on technical advancements that compromise environmental integrity, in order to safeguard the overall quality of the environment. The government should formulate requisite policies to promote low-interest loans for efficient technology. This initiative will enhance the technological capabilities in the selected countries, potentially resulting in a decrease in resource utilization. Technological innovation may be sustained in economies that are heavily polluted, and its progress can be accelerated by increasing investment in research and development. Supporting investment in technology can be achieved through the provision of tax incentives and subsidies.

The aforementioned conclusions carry significant policy consequences. First and foremost, investing in environment-related technology (ERT) helps to reduce the ecological imprint. Hence, governments should propose policies that incentivize investors to invest in Environmental Remediation Technologies (ERT) in polluted economies in order to mitigate environmental degradation. This measure is expected to be advantageous for these economies as they are now in a developmental phase, and their investment in technology will ultimately guide their future trajectory. Therefore, the choice to invest in Emission Reduction Technologies (ERTs) has the potential to yield favorable financial consequences and contribute to the attainment of SDG’s. Furthermore, this study posited that implementing supportive policies for ERT advancement in the chosen nations could expedite the lowering of EFP. Thus, it is imperative for governments to encourage investment in ERT (Energy Research and Technology) to bolster the clean energy industry and actively engage in the transition towards sustainable energy sources. It is recommended that governments provide incentives to private investors to capitalize on ERT (Environmental Remediation Technologies) and establish worldwide technological collaborations to mitigate global and regional environmental issues.

From the results, we have deduced various significant policy implications. Financial inclusion can serve as a requirement to attract private investment for low-carbon projects. In order for financial services to utilize private investment, it is necessary to first construct the financial infrastructure. This research demonstrated how important it is for banks to encourage new ideas like green credit guarantee schemes (GCGSs) and the spillover effect of taxes in order to attract private investment while decreasing risk. Governments in filthy economies should increase access to credit, which will encourage the growth of the financial sector and the recruitment of new organizations to meet the increasing need for financial services. In addition, governments should examine the different impacts of financial inclusion while establishing a regulatory structure that promotes a reliable and comprehensive financial system, so as to successfully combat the damage done to the environment. Furthermore, it is imperative to motivate consumers to improve their financial literacy in order to effectively utilize the existing financial services. Furthermore, it is crucial for policy makers and regulators to recognize and address concerns pertaining to financial regulation, inclusion, and development, as these issues are directly relevant to the implementation of policies aimed at mitigating carbon emissions. Therefore, it is imperative for each government to establish a comprehensive green funding program in order to attain the 2030 SDG’s of carbon neutrality and environmental sustainability. Furthermore, it is imperative for authorities in these economies to embrace and execute strategies to mitigate the situation.

The present study indicates that shifting investment from fossil fuel energy to RNE sources could yield sustainable outcomes, including a decrease in ecological impact and the attainment of cost-effectiveness, profitability, and minimal externalities. Developing countries typically rely on fossil fuels as their conventional energy sources. Nevertheless, this choice proved to be a double-edged sword since fossil fuel energy not only contributes to environmental pollution but also leads to rising manufacturing expenses. This condition implies that the utilization of RNE is advantageous in both the short and long term. Hence, it is suggested that energy authorities encourage investments in RNE inside economies that are heavily polluted. Regarding this matter, the conventional reliance on fossil fuels Countries with economies that are heavily polluted should incorporate a greater proportion of renewable resources into their energy mix. Nevertheless, due to the existing technological and infrastructural constraints, increasing the proportion of renewable energy in the overall energy consumption profile may pose a challenging endeavor for these countries. Hence, in addition to augmenting the utilization of renewable energy, it is imperative to substitute conventional fossil fuels with comparably cleaner alternatives. These fuels are likely to serve as temporary fuels until these countries can overcome the obstacles that have hindered the growth of renewable energy industries in polluted economies.

The empirical results we obtained strongly support the policy implications, as they demonstrate that economic expansion plays a key role in influencing the quality of the environment. In order to ensure long-term EG and prevent environmental deterioration, it is advisable for countries with high levels of pollution to give priority to energy efficiency projects and allocate resources towards cleaner energy investments. To get there, dirty economies should push for the widespread use of RNE sources which involves wind, solar, and nuclear electricity for both residential and commercial use. Its goal is to reduce energy consumption’s negative impact on the environment by promoting the prudent use of limited resources. Additionally, it should lessen the EFP associated with green policies that try to lessen the overall damage to the environment. So, polluted economies must have a clear plan that balances economic growth with environmental degradation. Lastly, polluted economies must look closely at their energy subsidy programmers and tighten environmental regulations, especially for polluting companies. These rules can ease the load on the environment. The government could use the money to buy greener industrial gear and technology, protecting the environment.

The current analysis suggests that reallocating funds from fossil fuel energy to RNE sources could result in sustainable outcomes, such as reduced ecological impact and the achievement of cost-effectiveness, profitability, and minimum externalities. Developing nations commonly depend on fossil fuels as their primary energy sources. However, this decision has both positive and negative consequences as the use of fossil fuel energy not only adds to environmental degradation but also results in increased industrial costs. This situation suggests that the use of RNE is beneficial in both the short and long run. Hence, it is advised that energy authorities support investments in renewable energy inside economies that are badly polluted. Regarding this subject, the traditional dependence on fossil fuels Nations with economies that experience significant pollution should integrate a higher percentage of renewable resources into their energy portfolio. However, the countries may have difficulties in increasing the share of renewable energy in their overall energy consumption profile due to existing technological and infrastructure limitations. Therefore, it is crucial to replace traditional fossil fuels with cleaner alternatives in order to further increase the use of RNE. These fuels are expected to function as interim energy sources until these nations can surmount the barriers that have impeded the development of RNE sectors in environmentally degraded economies.

The empirical findings we acquired robustly endorse the policy implications, as they illustrate that economic growth significantly influences the environmental quality. To promote sustainable EG and mitigate environmental degradation, countries with significant pollution levels should prioritize energy efficiency initiatives and direct resources towards investments in cleaner energy sources. To achieve this objective, polluting economies should promote the usage of renewable energy sources in both production as well as consumption, including nuclear power, solar power, and wind power. To lessen the damage that utilization of energy does to the environment, we must encourage the wise use of our finite resources. It should also decrease the EFP associated with the execution of environmentally-conscious policies aimed at reducing total environmental damage. Hence, it is imperative for economies grappling with pollution to adopt a clearly defined and all-encompassing policy that strikes a harmonious equilibrium between economic progress and environmental deterioration. To tackle pollution concerns, economies ought to undertake a thorough assessment of their energy subsidy initiatives and strengthen environmental laws, with a particular focus on organizations that make substantial contributions to the pollution predicament. These regulations can alleviate the environmental burden. The government could grant funding for the procurement of eco-friendly cutting-edge technology and manufacturing equipment, so ensuring the preservation of environmental integrity.

## Abbreviations

SDGs: Sustainable Development Goals
GW: Giga Watt
CO_2_: Carbon emissions
GHG: Greenhouse Gas emissions
EFP: Ecological Footprint
EKC: Environmental Kuznets Curve hypothesis
GDP: Gross Domestic Product
EE: Energy Efficiency
TECH: Technological advancement
OECD: Organization of Economic Cooperation and Development
REC: Renewable energy consumption
CT: Climate technology
FIN: Financial Inclusion
EG: Economic growth
CSD: Cross-Sectional Dependence
SH: Slope of homogeneity
CS-ARDL: Cross Sectional Autoregression Distribution test
DH Causality: CCE-MG: Common Correlated Effect mean Group
AMG: Augmented Mean Group

## References

[1] LiuZ.; VuT.L.; PhanT.T.H.; NgoT.Q.; AnhN.H.V.; PutraA.R.S. Financial Inclusion and Green Economic Performance for Energy Efficiency Finance. Econ. Chang. Restruct. 2022, 1–31, doi: 10.1007/s10644-022-09393-5

[2] VoD.H.; NguyenN.T.; Thi-Hong VanL. Financial Inclusion and Stability in the Asian Region Using Bank-Level Data. Borsa Istanbul Rev. 2021, 21, 36–43, 10.1016/j.bir.2020.06.003.

[3] FareedZ.; RehmanM.A.; AdebayoT.S.; WangY.; AhmadM.; ShahzadF. Financial Inclusion and the Environmental Deterioration in Eurozone: The Moderating Role of Innovation Activity. Technol. Soc. 2022, 69, 101961, doi: 10.1016/j.techsoc.2022.101961

[4] MehmoodU. Examining the Role of Financial Inclusion towards CO2 Emissions: Presenting the Role of Renewable Energy and Globalization in the Context of EKC. Environ. Sci. Pollut. Res. 2021, doi: 10.1007/s11356-021-16898-5 34633617

[5] RenzhiN.; BaekY.J. Can Financial Inclusion Be an Effective Mitigation Measure? Evidence from Panel Data Analysis of the Environmental Kuznets Curve. Financ. Res. Lett. 2020, 37, 101725, 10.1016/j.frl.2020.101725.

[6] HassanT.; SongH.; KhanY.; KirikkaleliD. Energy Efficiency a Source of Low Carbon Energy Sources? Evidence from 16 High-Income OECD Economies. Energy 2022, 243, 123063, doi: 10.1016/j.energy.2021.123063

[7] NietoJ.; CarpinteroÓ.; MiguelL.J. Less than 2°C? An Economic-Environmental Evaluation of the Paris Agreement. Ecol. Econ. 2018, 146, 69–84, doi: 10.1016/j.ecolecon.2017.10.007

[8] GrohmannA.; KlühsT.; MenkhoffL. Does Financial Literacy Improve Financial Inclusion? Cross Country Evidence. World Dev. 2018, 111, 84–96, doi: 10.1016/J.WORLDDEV.2018.06.020

[9] AzamA.; RafiqM.; ShafiqueM.; YuanJ. Mitigating Carbon Emissions in China: The Role of Clean Energy, Technological Innovation, and Political-Institutional Quality. Front. Environ. Sci. 2022, 10, 814439, doi: 10.3389/FENVS.2022.814439/BIBTEX

[10] FengH.; LiuZ.; WuJ.; IqbalW.; AhmadW.; MarieM. Nexus between Government Spending’s and Green Economic Performance: Role of Green Finance and Structure Effect. Environ. Technol. Innov. 2022, 27, 102461, doi: 10.1016/j.eti.2022.102461

[11] KesickiF.; AnandarajahG. The Role of Energy-Service Demand Reduction in Global Climate Change Mitigation: Combining Energy Modelling and Decomposition Analysis. Energy Policy 2011, 39, 7224–7233, doi: 10.1016/j.enpol.2011.08.043

[12] KumariS.; HarikrishnanA. Importance of Financial Literacy For Sustainable Future Environment: A Research Among People In Rural Areas With Special Reference To Mandi District,Himachal Pradesh. Int. J. Eng. Sci. Inf. Technol. 2021, 1, 15–19, doi: 10.52088/ijesty.v1i1.36

[13] OnifadeS.T.; AlolaA.A. Energy Transition and Environmental Quality Prospects in Leading Emerging Economies: The Role of Environmental‐related Technological Innovation. Sustain. Dev. 2022, doi: 10.1002/sd.2346

[14] GeddesA.; SchmidN.; SchmidtT.S.; SteffenB. The Politics of Climate Finance: Consensus and Partisanship in Designing Green State Investment Banks in the United Kingdom and Australia. Energy Res. Soc. Sci. 2020, 69, 101583, 10.1016/j.erss.2020.101583.

[15] LiuH.; AnwarA.; RazzaqA.; YangL. The Key Role of Renewable Energy Consumption, Technological Innovation and Institutional Quality in Formulating the SDG Policies for Emerging Economies: Evidence from Quantile Regression. Energy Reports 2022, 8, 11810–11824, doi: 10.1016/J.EGYR.2022.08.231

[16] GuptaM.; SainiS.; SahooM. Determinants of Ecological Footprint and PM2.5: Role of Urbanization, Natural Resources and Technological Innovation. Environ. Challenges 2022, 7, 100467, doi: 10.1016/j.envc.2022.100467

[17] BashirM.F.; MAB.; BashirM.A.; RadulescuM.; ShahzadU. Investigating the Role of Environmental Taxes and Regulations for Renewable Energy Consumption: Evidence from Developed Economies. Econ. Res. Istraz. 2022, 35, 1262–1284, doi: 10.1080/1331677X.2021.1962383

[18] JahangerA.; OzturkI.; Chukwuma OnweJ.; JosephT.E.; Razib HossainM. Do Technology and Renewable Energy Contribute to Energy Efficiency and Carbon Neutrality? Evidence from Top Ten Manufacturing Countries. Sustain. Energy Technol. Assessments 2023, 56, 103084, doi: 10.1016/J.SETA.2023.103084

[19] SadiqM.; ShinwariR.; UsmanM.; OzturkI.; MaghyerehA.I. Linking Nuclear Energy, Human Development and Carbon Emission in BRICS Region: Do External Debt and Financial Globalization Protect the Environment? Nucl. Eng. Technol. 2022, 54, 3299–3309, doi: 10.1016/J.NET.2022.03.024

[20] KnopfB.; ChenY.H.H.; De CianE.; FörsterH.; KanudiaA.; KarkatsouliI.; et al. BEYOND 2020-STRATEGIES and COSTS for TRANSFORMING the EUROPEAN ENERGY SYSTEM. Clim. Chang. Econ. 2013, doi: 10.1142/S2010007813400010

[21] UllahS.; AliK.; ShahS.A.; EhsanM. Environmental Concerns of Financial Inclusion and Economic Policy Uncertainty in the Era of Globalization: Evidence from Low & High Globalized OECD Economies. Environ. Sci. Pollut. Res. 2022, 1, 1–15, doi: 10.1007/s11356-022-18758-2 35064882 PMC8783182

[22] ZaidiS.A.H.; HussainM.; Uz ZamanQ. Dynamic Linkages between Financial Inclusion and Carbon Emissions: Evidence from Selected OECD Countries. Resour. Environ. Sustain. 2021, 4, 100022, doi: 10.1016/j.resenv.2021.100022

[23] MuafueshianghaI.M. The Impact of Financial Inclusion on Agricultural Development in Ngoketunjia Division, North West Cameroon. Swiss Sch. Bus. Manag. Geneva 2021, 5–24.

[24] LiN.; PeiX.; HuangY.; QiaoJ.; ZhangY.; HussainR. Impact of Financial Inclusion and Green Bond Financing for Renewable Energy Mix: Implications for Financial Development in OECD Economies. 2021, doi: 10.1007/s11356-021-17561-9 34843047 PMC8628031

[25] KoomsonI.; DanquahM. Financial Inclusion and Energy Poverty: Empirical Evidence from Ghana. Energy Econ. 2021, 94, 105085, 10.1016/j.eneco.2020.105085.

[26] AmariM.; AnisJ. Exploring the Impact of Socio-Demographic Characteristics on Financial Inclusion: Empirical Evidence from Tunisia. Int. J. Soc. Econ. 2021, 48, 1331–1346, doi: 10.1108/IJSE-08-2020-0527

[27] KaraA.; ZhouH.; ZhouY. Achieving the United Nations’ Sustainable Development Goals through Financial Inclusion: A Systematic Literature Review of Access to Finance across the Globe. Int. Rev. Financ. Anal. 2021, 77, 101833, 10.1016/j.irfa.2021.101833.

[28] LiuH.; YaoP.; LatifS.; AslamS.; IqbalN. Impact of Green Financing, FinTech, and Financial Inclusion on Energy Efficiency. Environ. Sci. Pollut. Res. 2022, 29, 18955–18966, doi: 10.1007/s11356-021-16949-x 34705207 PMC8548854

[29] KebedeJ.; SelvanathanS.; NaranpanawaA. Foreign Bank Presence, Institutional Quality, and Financial Inclusion: Evidence from Africa. Econ. Model. 2021, 102, 105572, 10.1016/j.econmod.2021.105572.

[30] WangL.; WangY.; SunY.; HanK.; ChenY. Financial Inclusion and Green Economic Efficiency: Evidence from China. J. Environ. Plan. Manag. 2022, 65, 240–271, doi: 10.1080/09640568.2021.1881459

[31] BurchiA.; WłodarczykB.; SzturoM.; MartelliD. The Effects of Financial Literacy on Sustainable Entrepreneurship. Sustain. 2021, 13.

[32] CaiX.; WeiC. Does Financial Inclusion and Renewable Energy Impede Environmental Quality: Empirical Evidence from BRI Countries. Renew. Energy 2023, 209, 481–490, doi: 10.1016/J.RENENE.2023.04.009

[33] LuoY.; PengY.; ZengL. Digital Financial Capability and Entrepreneurial Performance. Int. Rev. Econ. Financ. 2021, 76, 55–74, 10.1016/j.iref.2021.05.010.

[34] NaorM.; PintoG.D.; DavidovP.; BenarochJ.; KivelA. Inclusion of Ultra-Orthodox Students in Higher Education: A Case Study about Women Seminary in the Engineering College of Jerusalem. Educ. Sci. 2022, Vol. 12, Page 102 2022, 12, 102, doi: 10.3390/EDUCSCI12020102

[35] BannaH.; Kabir HassanM.; RashidM. Fintech-Based Financial Inclusion and Bank Risk-Taking: Evidence from OIC Countries. J. Int. Financ. Mark. Institutions Money 2021, 75, 101447, 10.1016/j.intfin.2021.101447.

[36] ChucA.T.; LiW.; PhiN.T.M.; LeQ.T.; YoshinoN.; Taghizadeh-HesaryF. The Necessity of Financial Inclusion for Enhancing the Economic Impacts of Remittances. Borsa Istanbul Rev. 2021, 10.1016/j.bir.2020.12.007.

[37] DuQ.; WuN.; ZhangF.; LeiY.; SaeedA. Impact of Financial Inclusion and Human Capital on Environmental Quality: Evidence from Emerging Economies. Environ. Sci. Pollut. Res. 2022, 1, 1–13, doi: 10.1007/s11356-021-17945-x 35025039

[38] OjoT.A. Financial Inclusion and Women Empowerment in BRICS Countries: Perspectives on India and South Africa. Int. Polit. Econ. Ser. 2022, 175–203, doi: 10.1007/978-3-030-97397-1_10/COVER

[39] EldeebM.S.; HalimY.T.; KamelE.M. The Pillars Determining Financial Inclusion among SMEs in Egypt: Service Awareness, Access and Usage Metrics and Macroeconomic Policies. Futur. Bus. J. 2021, doi: 10.1186/s43093-021-00073-w

[40] MenkehM.I. THE IMPACT OF FINANCIAL INCLUSION ON AGRICULTURAL DEVELOPMENT IN NGOKETUNJIA DIVISION, NORTH WEST CAMEROON. 2021.

[41] TsimisarakaR.S.M.; XiangL.; AndrianarivoA.R.N.A.; JosoaE.Z.; KhanN.; HanifM.S.; et al. Impact of Financial Inclusion, Globalization, Renewable Energy, ICT, and Economic Growth on CO2 Emission in OBOR Countries. Sustain. 2023, Vol. 15, Page 6534 2023, 15, 6534, doi: 10.3390/SU15086534

[42] AhmadM.; AhmedZ.; BaiY.; QiaoG.; PoppJ.; OláhJ. Financial Inclusion, Technological Innovations, and Environmental Quality: Analyzing the Role of Green Openness. Front. Environ. Sci. 2022, 10, 80, doi: 10.3389/fenvs.2022.851263

[43] KoomsonI.; VillanoR.A.; HadleyD. Effect of Financial Inclusion on Poverty and Vulnerability to Poverty: Evidence Using a Multidimensional Measure of Financial Inclusion. Soc. Indic. Res. 2020, 149, 613–639, doi: 10.1007/S11205-019-02263-0/TABLES/6

[44] BaskayaM.M.; Samour; * -TursoyA. THE FINANCIAL INCLUSION, RENEWABLE ENERGY AND CO2 EMISSIONS NEXUS IN THE BRICS NATIONS: NEW EVIDENCE BASED ON THE METHOD OF MOMENTS QUANTILE REGRESSION. 2022, doi: 10.15666/aeer/2003_25772595

[45] LeT.H.; LeH.C.; Taghizadeh-HesaryF. Does Financial Inclusion Impact CO2 Emissions? Evidence from Asia. Financ. Res. Lett. 2020, 34, 101451, doi: 10.1016/j.frl.2020.101451

[46] JiaS.; QiuY.; YangC. Sustainable Development Goals, Financial Inclusion, and Grain Security Efficiency. Agronomy 2021, 11, doi: 10.3390/AGRONOMY11122542

[47] EtonM.; MwosiF.; EjangM. The Effect of COVID-19 on Financial Inclusion in the Kigezi and Lango Subregions in Uganda. 10.1080/26437015.2021.1991859 2022, 1–14

[48] WeiminZ.; Sibt-e-AliM.; TariqM.; DagarV.; KhanM.K. Globalization toward Environmental Sustainability and Electricity Consumption to Environmental Degradation: Does EKC Inverted U-Shaped Hypothesis Exist between Squared Economic Growth and CO2 Emissions in Top Globalized Economies. Environ. Sci. Pollut. Res. 2022, 29, 59974–59984, doi: 10.1007/s11356-022-20192-3 35412186

[49] NingQ.Q.; GuoS.L.; ChangX.C. Nexus between Green Financing, Economic Risk, Political Risk and Environment: Evidence from China. Econ. Res. Istraz. 2021, 1–25, doi: 10.1080/1331677X.2021.2012710

[50] AhmadM.; JabeenG. Dynamic Causality among Urban Agglomeration, Electricity Consumption, Construction Industry, and Economic Performance: Generalized Method of Moments Approach. Environ. Sci. Pollut. Res. 2020, 27, 2374–2385, doi: 10.1007/s11356-019-06905-1 31782096

[51] KhanM.K.; TengJ.Z.; KhanM.I.; KhanM.O. Impact of Globalization, Economic Factors and Energy Consumption on CO2 Emissions in Pakistan. Sci. Total Environ. 2019, 688, 424–436, doi: 10.1016/j.scitotenv.2019.06.065 31247484

[52] AlvaradoR.; TillaguangoB.; DagarV.; AhmadM.; IşıkC.; MéndezP.; ToledoE. Ecological Footprint, Economic Complexity and Natural Resources Rents in Latin America: Empirical Evidence Using Quantile Regressions. J. Clean. Prod. 2021, 318, 128585, doi: 10.1016/J.JCLEPRO.2021.128585

[53] AdedoyinF.F.; OzturkI.; AgboolaM.O.; AgboolaP.O.; BekunF.V. The Implications of Renewable and Non-Renewable Energy Generating in Sub-Saharan Africa: The Role of Economic Policy Uncertainties. Energy Policy 2021, 150, 112115, doi: 10.1016/j.enpol.2020.112115

[54] WangQ.; ZhangF. What Does the China’s Economic Recovery after COVID-19 Pandemic Mean for the Economic Growth and Energy Consumption of Other Countries? J. Clean. Prod. 2021, 295, 126265, doi: 10.1016/j.jclepro.2021.126265 33589853 PMC7874931

[55] BurgerP.; CalitzE. Covid-19, Economic Growth and South African Fiscal Policy. South African J. Econ. 2021, 89, 3–24, doi: 10.1111/saje.12270

[56] CaoJ.; LawS.H.; SamadA.R.B.A.; MohamadW.N.B.W.; WangJ.; YangX. Impact of Financial Development and Technological Innovation on the Volatility of Green Growth—Evidence from China. Environ. Sci. Pollut. Res. 2021, 28, 48053–48069, doi: 10.1007/s11356-021-13828-3 33904131

[57] ZhaoX.; MaX.; ShangY.; YangZ.; ShahzadU. Green Economic Growth and Its Inherent Driving Factors in Chinese Cities: Based on the Metafrontier-Global-SBM Super-Efficiency DEA Model. Gondwana Res. 2022, 106, 315–328, doi: 10.1016/J.GR.2022.01.013

[58] KhanH.; WeiliL.; KhanI.; ZhangJ. The Nexus between Natural Resources, Renewable Energy Consumption, Economic Growth, and Carbon Dioxide Emission in BRI Countries. Environ. Sci. Pollut. Res. 2023, 30, 36692–36709, doi: 10.1007/s11356-022-24193-0 36562975

[59] DíazA.; MarreroG.A.; PuchL.A.; RodríguezJ. Economic Growth, Energy Intensity and the Energy Mix. Energy Econ. 2019, 81, 1056–1077, 10.1016/j.eneco.2019.05.022.

[60] KhowajaI.A.; TalpurU.; SoomroS.H.; KhanM.S. The Non-Banking Financial Institutions in Perspective of Economic Growth of Pakistan. Appl. Econ. Lett. 2021, 28, 701–706, doi: 10.1080/13504851.2020.1771266

[61] RenS.; DuM.; BuW.; LinT. Assessing the Impact of Economic Growth Target Constraints on Environmental Pollution: Does Environmental Decentralization Matter? J. Environ. Manage. 2023, 336, 117618, doi: 10.1016/j.jenvman.2023.117618 36905691

[62] PavlovaM. Fostering Inclusive, Sustainable Economic Growth and ‘“Green”‘ Skills Development in Learning Cities through Partnerships. Int. Rev. Educ. 2018, 64, doi: 10.1007/s11159-018-9718-x

[63] MardaniA.; StreimikieneD.; CavallaroF.; LoganathanN.; KhoshnoudiM. Carbon Dioxide (CO2) Emissions and Economic Growth: A Systematic Review of Two Decades of Research from 1995 to 2017. Sci. Total Environ. 2019, 649, 31–49. doi: 10.1016/j.scitotenv.2018.08.229 30170214

[64] SalahuddinM.; GowJ.; OzturkI. Is the Long-Run Relationship between Economic Growth, Electricity Consumption, Carbon Dioxide Emissions and Financial Development in Gulf Cooperation Council Countries Robust? Renew. Sustain. Energy Rev. 2015, 51, 317–326.

[65] FuinhasJ.A.; KoengkanM.; FilipeR.; SantiagoB.; MadalenoM.; NogueiraM.C. How Renewable Energy and CO2 Emissions Contribute to Economic Growth, and Sustainability—An Extensive Analysis. Sustain. 2023, Vol. 15, Page 4089 2023, 15, 4089, doi: 10.3390/SU15054089

[66] RazzaqA.; SharifA.; NajmiA.; TsengM.L.; LimM.K. Dynamic and Causality Interrelationships from Municipal Solid Waste Recycling to Economic Growth, Carbon Emissions and Energy Efficiency Using a Novel Bootstrapping Autoregressive Distributed Lag. Resour. Conserv. Recycl. 2021, 166, 105372, doi: 10.1016/J.RESCONREC.2020.105372

[67] ShangY.; PuY.; YuY.; GaoN.; LuY. Role of the E-Exhibition Industry in the Green Growth of Businesses and Recovery. Econ. Chang. Restruct. 2023, 56, 2003–2020, doi: 10.1007/S10644-023-09502-Y/TABLES/6

[68] RehmanA.; ZhangD.; ChandioA.A.; IrfanM. Does Electricity Production from Different Sources in Pakistan Have Dominant Contribution to Economic Growth? Empirical Evidence from Long-Run and Short-Run Analysis. Electr. J. 2020, 33, doi: 10.1016/j.tej.2020.106717

[69] DoğanB.; DrihaO.M.; Balsalobre LorenteD.; ShahzadU. The Mitigating Effects of Economic Complexity and Renewable Energy on Carbon Emissions in Developed Countries. Sustain. Dev. 2021, 29, 1–12, doi: 10.1002/sd.2125

[70] AliS.A.; AlharthiM.; HussainH.I.; RasulF.; HanifI.; HaiderJ.; UllahS.; ur RahmanS.; AbbasQ. A Clean Technological Innovation and Eco-Efficiency Enhancement: A Multi-Index Assessment of Sustainable Economic and Environmental Management. Technol. Forecast. Soc. Change 2021, 166, 120573, doi: 10.1016/J.TECHFORE.2021.120573

[71] JabeenA.; KhanS.A. Economic Growth, Social Inclusion, and Environmental Protection: Assessing the Existence of Green Growth in Pakistan. Environ. Sci. Pollut. Res. 2022, 29, doi: 10.1007/s11356-022-20467-9 35504994

[72] Mendoza-Del VillarL.; Oliva-LopezE.; Luis-PinedaO.; BenešováA.; TupaJ.; Garza-ReyesJ.A. Fostering Economic Growth, Social Inclusion & Sustainability in Industry 4.0: A Systemic Approach. In Proceedings of the Procedia Manufacturing; 2020; Vol. 51.

[73] HuJ.L.; ChenY.C.; YangY.P. The Development and Issues of Energy-ICT: A Review of Literature with Economic and Managerial Viewpoints. Energies 2022, Vol. 15, Page 594 2022, 15, 594, doi: 10.3390/EN15020594

[74] TangC.F.; TanB.W.; OzturkI. Energy Consumption and Economic Growth in Vietnam. Renew. Sustain. Energy Rev. 2016.

[75] SamargandiN.; KutanA.M.; SohagK.; AlqahtaniF. Equity Market and Money Supply Spillovers and Economic Growth in BRICS Economies: A Global Vector Autoregressive Approach. North Am. J. Econ. Financ. 2020, 51, doi: 10.1016/j.najef.2019.101060

[76] TonguraiJ.; VithessonthiC. The Impact of the Banking Sector on Economic Structure and Growth. Int. Rev. Financ. Anal. 2018, doi: 10.1016/j.irfa.2018.01.002

[77] SalariM.; JavidR.J.; NoghanibehambariH. The Nexus between CO2 Emissions, Energy Consumption, and Economic Growth in the U.S. Econ. Anal. Policy 2021, 69, 182–194, doi: 10.1016/j.eap.2020.12.007

[78] TariqG.; SunH.; Fernandez-GamizU.; MansoorS.; PashaA.A.; AliS.; et al. Effects of Globalization, Foreign Direct Investment and Economic Growth on Renewable Electricity Consumption. Heliyon 2023, 9, 2405–8440, doi: 10.1016/j.heliyon.2023.e14635 36994385 PMC10040718

[79] IsikC.; DogruT.; TurkE.S. A Nexus of Linear and Non-Linear Relationships between Tourism Demand, Renewable Energy Consumption, and Economic Growth: Theory and Evidence. Int. J. Tour. Res. 2018, 20, 38–49, doi: 10.1002/JTR.2151

[80] ZainalM.; Bani-MustafaA.; AlameenM.; ToglawS.; MazariA. Al Economic Anxiety and the Performance of SMEs during COVID-19: A Cross-National Study in Kuwait. Sustain. 2022, Vol. 14, Page 1112 2022, 14, 1112, doi: 10.3390/SU14031112

[81] PurnamawatiI.G.A. Sustainable Finance for Promoting Inclusive Growth. J. Ilm. Akunt. 2022, 6, 435, doi: 10.23887/jia.v6i2.39208

[82] ZhaoL.; ChauK.Y.; TranT.K.; SadiqM.; XuyenN.T.M.; PhanT.T.H. Enhancing Green Economic Recovery through Green Bonds Financing and Energy Efficiency Investments. Econ. Anal. Policy 2022, 76, 488–501, doi: 10.1016/j.eap.2022.08.019

[83] Aurangzaib; FarooqF. How Does Institutional Quality Moderates the Impact of Public Debt on Economic Growth? Startling Evidence from OIC Countries. Int. J. Manag. Res. Emerg. Sci. 2022, 12, doi: 10.56536/IJMRES.V12I3.287

[84] GwaniA.A.; SekS.K. Dynamic Modelling of Renewable Energy Consumption and Production on African Economic Growth and the Environment Using Vector Error Correction Models. Mat. Malaysian J. Ind. Appl. Math. 2023, 39, 15–31.

[85] HundieS.K. Income Inequality, Economic Growth and Carbon Dioxide Emissions Nexus: Empirical Evidence from Ethiopia. Environ. Sci. Pollut. Res. 2021, 28, 43579–43598, doi: 10.1007/s11356-021-13341-7 33840023

[86] PesaranM.H.; SmithR. The Role of Theory in Econometrics. J. Econom. 1995, 67, 61–79, doi: 10.1016/0304-4076(94)01627-C

[87] YangJ.; RizviS.K.A.; TanZ.; UmarM.; KoondharM.A. The Competing Role of Natural Gas and Oil as Fossil Fuel and the Non-Linear Dynamics of Resource Curse in Russia. Resour. Policy 2021, 72, doi: 10.1016/j.resourpol.2021.102100

[88] LiuD.; XieY.; HafeezM.; UsmanA. The Trade ‑ off between Economic Performance and Environmental Quality: Does Financial Inclusion Matter for Emerging Asian Economies? Environ. Sci. Pollut. Res. 2021, doi: 10.1007/s11356-021-17755-1 34993792

[89] PradhanR.P.; ArvinM.B.; NairM.S.; HallJ.H.; BennettS.E. Sustainable Economic Development in India: The Dynamics between Financial Inclusion, ICT Development, and Economic Growth. Technol. Forecast. Soc. Change 2021, 169, 120758, doi: 10.1016/J.TECHFORE.2021.120758

[90] HuangR.; KaleS.; ParamatiS.R.; Taghizadeh-HesaryF. The Nexus between Financial Inclusion and Economic Development: Comparison of Old and New EU Member Countries. Econ. Anal. Policy 2021, 69, 1–15, doi: 10.1016/j.eap.2020.10.007

[91] WuB.; LiuZ.; GuQ.; TsaiF.S. Underdog Mentality, Identity Discrimination and Access to Peer-to-Peer Lending Market: Exploring Effects of Digital Authentication. J. Int. Financ. Mark. Institutions Money 2023, 83, 101714, doi: 10.1016/J.INTFIN.2022.101714

[92] UddinM.N. Role of Islamic Microfinance Institutions for Sustainable Development Goals in Bangladesh. J. Int. Bus. Manag. 2020, doi: 10.37227/jibm-2020-64

[93] KassiD.F.; SunG.; DingN. Does Governance Quality Moderate the Finance-Renewable Energy-Growth Nexus? Evidence from Five Major Regions in the World. Environ. Sci. Pollut. Res. 2020, 27, 12152–12180, doi: 10.1007/s11356-020-07716-5 31989502

[94] GattoA.; Sadik-ZadaE.R. Access to Microfinance as a Resilience Policy to Address Sustainable Development Goals: A Content Analysis. Heliyon 2022, 8, doi: 10.1016/j.heliyon.2022.e10860 36267370 PMC9578961

[95] JiangY.; SharifA.; AnwarA.; The CongP.; LelchumananB.; Thi YenV.; et al. Does Green Growth in E-7 Countries Depend on Economic Policy Uncertainty, Institutional Quality, and Renewable Energy? Evidence from Quantile-Based Regression. Geosci. Front. 2023, 14, 101652, doi: 10.1016/J.GSF.2023.101652

[96] ChaudhryI.S.; YusopZ.; HabibullahM.S. Financial Inclusion-Environmental Degradation Nexus in OIC Countries: New Evidence from Environmental Kuznets Curve Using DCCE Approach. 2022, 5360–5377.10.1007/s11356-021-15941-934417974

[97] NanS.; HuangJ.; WuJ.; LiC. Does Globalization Change the Renewable Energy Consumption and CO2 Emissions Nexus for OECD Countries? New Evidence Based on the Nonlinear PSTR Model. Energy Strateg. Rev. 2022, 44, doi: 10.1016/j.esr.2022.100995

[98] SunY.; LiH.; ZhangK.; KamranH.W. Dynamic and Casual Association between Green Investment, Clean Energy and Environmental Sustainability Using Advance Quantile A.R.D.L. Framework. Econ. Res. Istraz. 2022, 35, 3609–3628, doi: 10.1080/1331677X.2021.1997627

[99] ChishtiM.Z.; SinhaA. Do the Shocks in Technological and Financial Innovation Influence the Environmental Quality? Evidence from BRICS Economies. Technol. Soc. 2022, 68, 101828, doi: 10.1016/j.techsoc.2021.101828

[100] QinL. Does Financial Inclusion Limit Carbon Dioxide Emissions? Analyzing the Role of Globalization and Renewable Electricity Output. 2021, 1138–1154, doi: 10.1002/sd.2208

[101] PataU.K.; KartalM.T. Impact of Nuclear and Renewable Energy Sources on Environment Quality: Testing the EKC and LCC Hypotheses for South Korea. Nucl. Eng. Technol. 2023, 55, 587–594, doi: 10.1016/J.NET.2022.10.027

[102] LepitzkiJ.; AxsenJ. The Role of a Low Carbon Fuel Standard in Achieving Long-Term GHG Reduction Targets. Energy Policy 2018, 119, 423–440, doi: 10.1016/j.enpol.2018.03.067

[103] HuanY.; QamruzzamanM. Innovation-Led FDI Sustainability: Clarifying the Nexus between Financial Innovation, Technological Innovation, Environmental Innovation, and FDI in the BRIC Nations. Sustain. 2022, Vol. 14, Page 15732 2022, 14, 15732, doi: 10.3390/SU142315732

[104] HabibaU.; XinbangC. The Impact of Financial Development on CO2 Emissions: New Evidence from Developed and Emerging Countries. Environ. Sci. Pollut. Res. 2022, doi: 10.1007/s11356-022-18533-3 35006573

[105] KetuS.; MishraP.K. Internet of Healthcare Things: A Contemporary Survey. J. Netw. Comput. Appl. 2021, 192, 103179, 10.1016/j.jnca.2021.103179.

[106] AdamsS.; AcheampongA.O. Reducing Carbon Emissions: The Role of Renewable Energy and Democracy. J. Clean. Prod. 2019, 240, 118245, doi: 10.1016/j.jclepro.2019.118245

[107] KhanS.A.R.; YuZ.; SharifA. No Silver Bullet for De-Carbonization: Preparing for Tomorrow, Today. Resour. Policy 2021, 71, 101942, doi: 10.1016/j.resourpol.2020.101942

[108] OforiE.K.; OnifadeS.T.; AliE.B.; AlolaA.A.; ZhangJ. Achieving Carbon Neutrality in Post COP26 in BRICS, MINT, and G7 Economies: The Role of Financial Development and Governance Indicators. J. Clean. Prod. 2023, 387, 135853, doi: 10.1016/J.JCLEPRO.2023.135853

[109] CapraM., La MottaS. International collaboration in climate technology innovation: the Italian experience in Mission Innovation. Sustain Sci 19, 203–206 (2024). 10.1007/s11625-023-01314-3.

[110] AbbasM.; ZainiA. Lecture Notes in Mechanical Engineering Proceedings of the 3rd International Conference on Separation Technology; 2021; ISBN 9789811607417.

[111] Anshika; SinglaA.; MallikG. Determinants of Financial Literacy: Empirical Evidence from Micro and Small Enterprises in India. Asia Pacific Manag. Rev. 2021, doi: 10.1016/j.apmrv.2021.03.001

[112] JuergensenJ.; GuimónJ.; NarulaR. European SMEs amidst the COVID-19 Crisis: Assessing Impact and Policy Responses. J. Ind. Bus. Econ. 2020, 47, 499–510, doi: 10.1007/s40812-020-00169-4

[113] KartikoN.D.; RachmiI.F. Pengaruh Net Profit Margin, Return On Asset, Return On Equity, Dan Earning Per Share Terhadap Harga Saham Di Masa Pandemi Covid-19 (Studi Empiris Pada Perusahaan Publik Sektor Pertambangan Di Bursa Efek Indonesia). J. Ris. Bisnis dan Investasi 2021, 7, 58–68, doi: 10.35313/jrbi.v7i2.2592

[114] Mendonça, A.K. de S.; de Andrade Conradi Barni, G.; Moro, M.F.; Bornia, A.C.; Kupek, E.; Fernandes, L. Hierarchical Modeling of the 50 Largest Economies to Verify the Impact of GDP, Population and Renewable Energy Generation in CO2 Emissions. Sustain. Prod. Consum. 2020, 22, 58–67, 10.1016/j.spc.2020.02.001.

[115] JianguoD.; AliK.; AlnoriF.; UllahS. The Nexus of Financial Development, Technological Innovation, Institutional Quality, and Environmental Quality: Evidence from OECD Economies. Environ. Sci. Pollut. Res. 2022 2938 2022, 29, 58179–58200, doi: 10.1007/s11356-022-19763-1 35362882 PMC8972663

[116] BreiM.; GadaneczB.; MehrotraA. SME Lending and Banking System Stability: Some Mechanisms at Work. Emerg. Mark. Rev. 2020, 43, 100676, 10.1016/j.ememar.2020.100676.

[117] ChenY.; kumaraE.K.; SivakumarV. Invesitigation of Finance Industry on Risk Awareness Model and Digital Economic Growth. Ann. Oper. Res. 2021, doi: 10.1007/s10479-021-04287-7

[118] YaoL.; YangX. Can Digital Finance Boost SME Innovation by Easing Financing Constraints?: Evidence from Chinese GEM-Listed Companies. PLoS One 2022, 17, e0264647, doi: 10.1371/journal.pone.0264647 35239717 PMC8893686

